# BRCA1 Regulates IFI16 Mediated Nuclear Innate Sensing of Herpes Viral DNA and Subsequent Induction of the Innate Inflammasome and Interferon-β Responses

**DOI:** 10.1371/journal.ppat.1005030

**Published:** 2015-06-29

**Authors:** Dipanjan Dutta, Sujoy Dutta, Mohanan Valiya Veettil, Arunava Roy, Mairaj Ahmed Ansari, Jawed Iqbal, Leela Chikoti, Binod Kumar, Karen E. Johnson, Bala Chandran

**Affiliations:** H. M. Bligh Cancer Research Laboratories, Department of Microbiology and Immunology, Chicago Medical School, Rosalind Franklin University of Medicine and Science, North Chicago, Illinois, United States of America; University of Southern California, UNITED STATES

## Abstract

The innate immune system pattern recognition receptors (PRR) are the first line of host defenses recognizing the various pathogen- or danger-associated molecular patterns and eliciting defenses by regulating the production of pro-inflammatory cytokines such as IL-1β, IL-18 or interferon β (IFN-β). NOD-like receptors (NLRs) and AIM2-like receptors (ALRs) are cytoplasmic inflammasome sensors of foreign molecules, including DNA. IFI16, a sequence-independent nuclear innate sensor ALR, recognizes episomal dsDNA genomes of herpes viruses such as KSHV, EBV, and HSV-1 in the infected cell nuclei, forms an inflammasome complex with ASC and procaspase1, and relocates into the cytoplasm leading into Caspase-1 and IL-1β generation. IFI16 also induces IFN-β during HSV-1 infection via the cytoplasmic STING-TBK1-IRF3 pathway. Thus far, whether IFI16 recognizes foreign DNA directly or utilizes other host protein(s) is unknown. Here, we demonstrate that BRCA1, a DNA damage repair sensor and transcription regulator, is in complex with IFI16 in the host cell nucleus, and their association increases in the presence of nuclear viral genomes during *de novo* KSHV, EBV and HSV-1 infection, and in latent KSHV or EBV infection, but not by DNA damage responses (DDR) induced by bleomycin and vaccinia virus cytoplasmic dsDNA. BRCA1 is a constituent of the triggered IFI16-inflammasome and is translocated into the cytoplasm after genome recognition along with the IFI16-inflammasome. The absence of BRCA1 abrogated IFI16-viral genome association, inflammasome assembly, IFI16 cytoplasmic localization, and Caspase-1 and IL-1β production. The absence of BRCA1 also abolished the cytoplasmic IFI16-STING interaction, downstream IRF3 phosphorylation, nuclear translocation of pIRF3 and IFN-β production during *de novo* KSHV and HSV-1 infection. These findings highlight that BRCA1 plays a hitherto unidentified innate immunomodulatory role by facilitating nuclear foreign DNA sensing by IFI16, subsequent assembly and cytoplasmic distribution of IFI16-inflammasomes leading into IL-1β formation and the induction of IFN-β via cytoplasmic signaling through IFI16-STING, TBK1 and IRF3.

## Author Summary

Invasion of a host cell by pathogens, including viruses, is sensed by pattern-recognition receptors resulting in the elicitation of the host innate defenses such as the formation of multi-protein inflammasome complexes, inflammatory IL-1β and IL-18 cytokine production and interferon-β production via the cytoplasmic STING molecule. We have shown that nuclear episomal viral DNA genomes of herpes viruses (KSHV, EBV and HSV-1) are sensed by the nuclear resident IFI16 protein, resulting in the formation of the IFI16-ASC-procaspase-1 inflammasome complex. Here, we show that BRCA1 promotes viral DNA sensing by IFI16 in the nucleus and is a constituent of the triggered IFI16-ASC-procaspase-1 inflammasome. IFI16 and BRCA1 are in complex in the nucleus and their association increases in the presence of KSHV, EBV or HSV-1 genomes, but not by the DNA damage response or vaccinia virus cytoplasmic dsDNA. The absence of BRCA1 results in abrogated IFI16-genome association, IFI16 cytoplasmic translocation, IL-1β production, IFI16 interaction with STING, IRF3 phosphorylation, pIRF3 nuclear translocation, and IFN-β induction. Taken together, these results demonstrate a crucial and novel role of BRCA1 in the innate sensing of viral DNA and subsequent induction of the inflammasome and interferon-β responses.

## Introduction

Sensing of microbial nucleic acids by pattern-recognition receptors (PRRs) is a crucial step for an effective innate immune response [1]. The best established function of PRRs like NLRPs (NOD-like receptors with PYRIN (PYD) domain) and ALRs (absent in melanoma 2 [AIM2]-like receptors) is their ability to sense pathogens and other danger signals. This leads into the formation of a multiprotein inflammasome complex consisting of a sensor protein, adaptor protein ASC (apoptosis-associated speck-like protein containing CARD) and procaspase-1 resulting in active Caspase-1 generation which cleaves the proforms of interleukin-1β (IL-1β), IL-18, and IL-33 cytokines.

Our studies have demonstrated that IFI16 (interferon inducible protein 16), a resident nuclear ALR protein in a variety of cells, functions as a sensor and detects nuclear replicating herpesvirus genomes such as Kaposi's sarcoma-associated herpesvirus (KSHV), Epstein-Barr virus (EBV), and herpes simplex virus type-1 (HSV-1) leading to IFI16-inflammasome formation [2, 3, 4, 5]. *De novo* KSHV infection of primary human microvascular dermal endothelial (HMVEC-d) cells and HSV-1 infection of primary human foreskin fibroblast (HFF) cells induces IFI16-ASC-procaspase-1 inflammasome formation in the nucleus and its redistribution to the cytoplasm [2, 5]. KSHV latency in endothelial and B cells also constitutively activates the IFI16-inflammasome and cytoplasmic relocalization, and IFI16 colocalizes with the KSHV and HSV-1 genomes in the nuclei of infected cells [2, 3]. EBV latency in B and epithelial cells also constitutively activates the IFI16 inflammasome and cytoplasmic relocalization, and IFI16 colocalizes with the EBV genomes in the nucleus [4].

IFI16 has also been shown to interact with STING (stimulator of interferon genes) leading to phosphorylation and nuclear translocation of IRF3 via the IFI16-STING-TBK signaling axis, resulting in IFN-β production during HSV-1 infection [6, 7]. The role of IFI16 as a silencing factor for the HSV-1 genome has also been reported [8]. We have also recently demonstrated that, independent of its innate immune response, IFI16 inhibited HSV-1 replication by repressing viral gene expression via its binding to the transcription start sites of viral genes, reducing the association of transcription factors to these sites and by promoting global histone modifications on the viral genome [9].

The linear epigenetically naïve virion-associated herpesviral dsDNA genome circularizes after entry into the nucleus, associates with histones and nucleosome proteins leading to epigenetic control [10, 11, 12]. The host cell DNA damage response (DDR) is a signal cascade event that includes the phosphorylation of repair mediators (H2AX, BRCA1, 53BP1, and Mdc1) and effectors of the checkpoint responses (CHK1 and CHK2). The DDR also recognizes exogenous genomes of nuclear DNA viruses which manipulate the DDR for their advantage [13]. Entry of KSHV DNA into the nuclei of endothelial cells during *de novo* infection induces an immediate DDR response of ATM kinase, H2AX and BRCA1 (breast cancer tumor suppressor protein) activation [14].

IFI16, believed to be a part of the large BRCA1-associated genome surveillance (BASC) DDR complex, interacts with BRCA1 and is implicated in BRCA1-mediated apoptosis and inflammation signaling [15]. IFI16 contains two DNA binding HIN domains, a transcriptional regulatory domain, an APIN/PAAD domain associated with the IFN response and an ASC binding PYD domain that also binds BRCA1 [16]. In a non-nuclear artificial system, IFI16 has been shown to bind to superhelical plasmid DNA and cruciform DNA [17]. A study suggested that IFI16 recognizes DNA in a non-sequence specific manner by electrostatic attraction between its positively charged HIN domain residues and the sugar-phosphate backbone of dsDNA [1]. However, questions such as whether pathogen DNA is recognized by IFI16 directly or in association with other host proteins and how IFI16 differentiates host vs. pathogen DNA remain unknown.

Here, we demonstrate that IFI16 is associated with BRCA1 in the nuclei of uninfected cells and that interaction increased during *de novo* KSHV and HSV-1 infection as well as during latent KSHV and EBV infection. Our studies show that BRCA1 is an essential component of the IFI16-inflammasome complex. In the absence of BRCA1, KSHV and HSV-1 genome recognition by IFI16, inflammasome complex formation and cytoplasmic localization, cleavage of caspase-1 and IL-1β, cytoplasmic association of IFI16 with STING, phosphorylation of IRF3, nuclear localization of pIRF3, and IFN-β production were abrogated. Collectively, these studies demonstrate that BRCA1 is a positive regulator of the foreign DNA sensing capability of IFI16 and a stabilizer of the IFI16 inflammasome complex and interferon responses.

## Results

### *De novo* KSHV infection enhances the interaction between IFI16 and DDR protein BRCA1 and IFI16 is not associated with DDR H2AX, CHK2 proteins

IFI16 forms a functional IFI16-ASC-procaspase-1 inflammasome early during *de novo* KSHV infection of primary HMVEC-d cells as well as in latently infected cells, and translocates to the cytoplasm [2, 3]. We have also observed the phosphorylation of ATM, H2AX, CHK2 and BRCA1, the key early DDR components, as soon as KSHV DNA enters the infected cell nuclei at 30 min post-infection (p.i.) [14]. Since IFI16 is suggested to be a part of the DDR [18, 19], we hypothesized that IFI16 forms complexes with different proteins to mediate different functions, and that one or more of these IFI16 complexes recognizes the KSHV DNA to induce inflammasomes.

To test this hypothesis, we utilized *de novo* KSHV infection that is well-characterized in our earlier studies [2, 3, 14] in which infected cells are identified by a variety of methods such as i) entry of KSHV into the cytoplasm measured by immunofluorescence assay (IFA) for viral envelope and capsid proteins or 5-bromo-2’-deoxyuridine (BrdU) or 5-ethynyl-2’-deoxyuridine (EdU) labeled KSHV genome, and ii) entry of viral DNA into the nucleus measured by IFA for BrdU or EdU and nuclear expression of viral latency associated LANA-1 protein by IFA [2, 3, 14]. In addition, relocalization of nuclear IFI16 into the cytoplasm is also considered as an indicator of infection [2, 3]. When HMVEC-d cells were infected with KSHV containing BrdU genome (30 DNA copies/cell) and immunostained with anti-BrdU antibodies (Table 1), several BrdU labeled viral particles (Fig 1A, green spots) were detected both in the cytoplasm as well as in the infected cell nucleus at 15 min (0.25h) p.i. (Fig 1A, white and yellow arrows, respectively). Similarly, when HFF cells were infected with KSHV containing EdU labeled viral genome (30 DNA copies/cell), we observed a gradual increase in nuclear entry of viral DNA from the cytoplasm during the observed 0.25 h, 0.5 h and 4 h p.i. (Fig 1B, arrows). When these cells were stained for IFI16, we observed the colocalization of IFI16 with the viral genomes in the nucleus (Fig 1C, panels 3 and 4). In addition, IFI16 was observed only in the cytoplasm of cells with nuclear-EdU KSHV genome (Fig 1C, white arrows) and not in the uninfected HFF cells. These observations also support our assertion that relocalization of nuclear IFI16 into the cytoplasm is an indication of KSHV infection. We utilized similar concentrations of labeled and unlabeled virus in all our experiments.

**Fig 1:** Enhanced interaction of IFI16 with BRCA1 but not with other DNA damage response proteins during *de novo* KSHV infection. **(A-C)** Analysis of *de novo* infection with BrdU or EdU genome labeled KSHV. (A) HMVEC-d cells were infected with BrdU genome labeled KSHV (30 DNA copies/cell) for 0.25 h and processed for IFA. Cells were fixed, permeabilized, treated with 4 N HCl and reacted with anti-BrdU antibodies followed by Alexa Fluor-488 secondary antibodies. Green spots represent BrdU KSHV genomes of representative virus infected cells. Yellow arrows: nuclear KSHV genome; white arrows: cytoplasmic KSHV genomes. (B) HFF cells uninfected or infected with EdU genome labeled virus for the indicated time points were processed for detection of EdU viral genome by Click-reaction with Alexa 594 labeled azide. Red spots and arrows indicate cytoplasmic or nuclear viral genome. Nuclei were stained with DAPI (blue). (C) Nuclear and cytoplasmic distribution of IFI16 during EdU KSHV infection (4 h p.i.) as shown in (B). HFF cells infected with EdU genome labeled KSHV (30 DNA copies/cell) were processed for IFA to detect IFI16 with anti-IFI16 antibodies followed by Alexa Fluor-488 secondary antibodies and then EdU labeled viral genomes were detected with Alexa 594 labeled azide by Click-reaction. Green staining represents IFI16; white arrows indicate cytoplasmic IFI16 in EdU (red) virus infected cells but not in uninfected cells. Nuclei were stained with DAPI (blue). **(D and E)** HMVEC-d cells infected with KSHV (30 DNA copies/cell) for 4 and 24 h. Lysates from uninfected (UI) and infected cells immunoprecipitated (IP-ed) with (D) anti-IFI16 and (E) BRCA1 antibodies and western blotted (WB) for BRCA1, IFI16, CHK2 and H2AX proteins. **(F)** Input controls for IP reactions in D and E. Whole cell-lysates (WCL) were blotted with anti-BRCA1, IFI16, CHK2, H2AX or β-actin antibodies. **(G)** Lysates from the above experiments (D and E) were used to IP with species specific IgG antibodies and WB for BRCA1, IFI16, CHK2 and H2AX for specificity controls (Ga). IP inputs were assessed by BRCA1, IFI16, CHK2, H2AX and β-actin WBs (Gb).

**Table 1:** List of antibodies used in this study.

Antibody	Species	Source
BRCA1	Mouse monoclonal	GeneTex, Irvine, CA
BRCA1	Rabbit polyclonal	Millipore Billerica, MA
H2AX, γH2AX	Rabbit monoclonal	Cell Signaling Technology, Beverly, MA
CHK2	Rabbit monoclonal	Cell Signaling Technology, Beverly, MA
ASC	Mouse monoclonal	MBL International, Woburn, MA
ASC/TMS1	Goat polyclonal	Ray Biotech, Norcross, GA
IL-1β	Mouse monoclonal	R&D Systems, Inc, Minneapolis, MN
IFI16	Mouse monoclonal, Goat polyclonal	Santa Cruz Biotechnology, Inc., Dallas, Texas
IFI16	Rabbit polyoclonal	Sigma, St Louis, MO
Caspase-1	Rabbit polyclonal	Bio Vision, Milpitas, CA
AIM2	Rabbit polyclonal	Abcam Inc., Cambridge, MA
NLRP3	Rabbit monoclonal	Abcam Inc., Cambridge, MA
STING	Rabbit monoclonal	Cell Signaling Technology, Beverly, MA
p-IRF3	Rabbit monoclonal	Cell Signaling Technology, Beverly, MA
IRF3	Mouse monoclonal	Abcam Inc., Cambridge, MA
β-actin	Mouse monoclonal	Sigma, St Louis, MO
β-tubulin	Mouse monoclonal	Sigma, St Louis, MO
TBP	Mouse monoclonal	Abcam Inc., Cambridge, MA
Histone H3	Rabbit monoclonal	Cell Signaling Technology, Beverly, MA
Alexa 488 and 594	Rabbit or Mouse	Molecular Probes, Invitrogen, Carlsbad, CA
Anti-rabbit-HRP and anti-mouse-HRP secondary		KPL Inc., Gaithersburg, MD

To determine whether IFI16 interacts with members of the DDR under physiological conditions, extracts from uninfected HMVEC-d cells or cells infected with KSHV for 4 and 24 h were immunoprecipitated (IP-ed) with anti-IFI16 antibody and western blotted for BRCA1, IFI16, CHK2 and H2AX. Compared to uninfected cells, we observed increased association of IFI16 with BRCA1 (~2.5 and ~4-fold at 4 and 24 h p.i., respectively) in the infected cells (Fig 1D, panel 1, lanes 1–4). In contrast, the interaction of IFI16 with CHK2 and H2AX proteins was not detected (Fig 1D, panels 3 and 4, lanes 1–4). To confirm these observations, the same extracts were IP-ed with anti-BRCA1 antibody and Western blotted for IFI16, BRCA1, CHK2 and H2AX. In these reactions we also observed an increased association of BRCA1 with IFI16 in infected cells (~ 3.1 and ~ 4.8 fold at 4 and 24 h p.i., respectively) compared with the uninfected cells (Fig 1E, panel 2, lanes 1–4). In contrast, we observed that BRCA1 interacted with CHK2 and H2AX similarly in both uninfected and infected cells without additional infection induced association (Fig 1E, panels 3 and 4, lanes 1–4). There were no overall changes in the total BRCA1, IFI16 and CHK2 levels except for the increase in H2AX levels as shown before [14] upon KSHV infection (Fig 1F, lanes 1–4). IP using control IgG showed no interaction with BRCA1, IFI16, CHK2 and H2AX (Fig 1Ga) with similar input levels of those proteins except increased H2AX in infected cell extracts (Fig 1Gb) as observed before [14] demonstrating the specificity of the reactions. These observations suggested that multiple complexes involving IFI16 and DDR proteins may be present under physiological conditions. However, IFI16 interacts with BRCA1 and not with CHK2 and H2AX proteins, and infection increases the BRCA1-IFI16 association.

The similar total protein level of cellular BRCA1 and IFI16 in both uninfected and virus infected cells as observed in the WB of input in Fig 1F and Fig 1Gb as well as in IP reactions shown in Fig 1D, panel 2 and Fig 1E, panel 1 imply that there are no overall changes in the expression of these proteins as a result of KSHV infection. However, our co-IP and reverse co-IP results (Fig 1D, panel 1 and Fig 1E, panel 2) show that compared to uninfected cells, increased co-IP of BRCA1 and IFI16 occur in the infected cells demonstrating that the increased association between IFI16 and BRCA1 is an infection induced phenomenon.

### Enhanced interaction between IFI16 and BRCA1 occur during *de novo* KSHV infection and not during DDR induction by bleomycin

To further assess that the observed increased interactions between IFI16 and BRCA1 are specifically due to viral infection in HMVEC-d cells, we studied the interactions between IFI16 and BRCA1 as well as interactions of H2AX and CHK2 with IFI16 and BRCA1 during bleomycin (10 mU/ml for 4 h) induced DDR and during KSHV infection. Under these conditions, increased levels of nuclear IFA spots representing phosphorylated H2AX (γH2AX), a well-established hallmark of DDR, were observed (Fig 2A, white arrows).

**Fig 2:** Proximity ligation assay and immunofluorescence microscopic analysis (IFA) of interactions and cellular distribution of complexes between IFI16, BRCA1, ChK2, γH2AX and ASC in untreated and bleomycin treated HMVEC-d cells. (**A**) Specificity of bleomycin action. HMVEC-d cells untreated and treated with bleomycin (10mU/ml) for 4 h. Cells were washed, fixed, permeabilized, blocked with signal enhancer (Image-IT), reacted with anti-γH2AX antibodies, washed and then incubated with Alexa 488 (green) conjugated secondary antibodies for IFA. Nuclei were stained using DAPI (blue). White box insets depict enlarged images. (**B and C**) Schematic diagram for PLA. This method detects endogenous protein interactions at spatial and subcellular resolution. PLA relies on the principle that if two epitopes of a single molecule such as molecule-A (B) or two molecules such as molecule-A and-B (C) are in the proximity of 40 nm or below, the species specific PLA oligo probes (minus and plus probes) linked to two secondary antibodies bound to primary antibody-antigen complexes get hybridized in the presence of 2 additional oligonucleotides to facilitate hybridization. Hybridized oligonucleotides are then ligated to form a closed circle, which serves as a template for rolling-circle amplification after adding an amplification solution with fluorescently labeled oligonucleotides to generate a concatemeric product extending from the oligonucleotide arm of the PLA probes. Fluorescently labeled oligonucleotides subsequently hybridized to the concatemeric products generate amplified signals which are detected as distinct fluorescent dots under fluorescence microscopy. **(D)** HMVEC-d cells untreated and uninfected (UI) or treated with bleomycin (10mU/ml) or infected with KSHV (30 DNA copies /cell) for 4 h. Cells were processed as described for (A) and reacted with the indicated pairs of primary antibodies followed by PLA to assess the interactions between IFI16 and BRCA1; BRCA1 and CHK2; BRCA1 and γH2AX; IFI16 and ASC; IFI16 and CHK2; and IFI16 and γH2AX. Nuclei were stained with DAPI. PLA reaction was detected using DUOLink green detection agent. White and yellow arrows: puncta in the nucleus or cytoplasm, respectively, indicating a positive PLA signal suggesting interactions among the two proteins. White box insets depict enlarged images. Quantitative analysis of the average number of IFI16+BRCA1 interaction PLA spots per cell is presented in the bottom bar graph. *: p<0.05.

We performed a proximity ligation assay (PLA) to study the interactions between IFI16 and DDR proteins. PLA can detect an endogenous individual protein or interactions of two proteins and their localization. It relies on the principle that if two epitopes/proteins are within the proximity of 40 nm or below, the PLA oligo probes linked to two secondary antibodies bound to primary antibody-antigen complexes will be amplified to give a PLA signal visualized as a fluorescent dot (Fig 2B and 2C). PLA of untreated and bleomycin treated cells was performed using only one primary antibody in combination with anti-rabbit MINUS probe and anti-mouse PLUS probe. The lack of detection of any PLA signals under all experimental conditions validated the specificity of the antibodies and observed reactions (S1 Fig).

We performed PLA to assess the respective protein-protein interactions using the following combinations of primary antibodies: IFI16+BRCA1, BRCA1+CHK2, BRCA1+γH2AX, IFI16+ASC, IFI16+CHK2, and IFI16+γH2AX (Fig 2D, S1 Table). ASC, a non-DDR protein, was included as a negative control. Bleomycin induced DDR led to increased nuclear interactions between BRCA1-CHK2 and BRCA1-γH2AX (Fig 2D, 2^nd^ row, 2^nd^ and 3^rd^ blocks, white arrows) and no such interaction was observed between IFI16 and ASC (Fig 2D, 2^nd^ row, 4th block). Interestingly, we observed similar levels of interactions between IFI16 and BRCA1 in both untreated and bleomycin treated cells (Fig 2D, 1^st^ and 2^nd^ rows, 1st block, white arrows). Furthermore, no interactions were observed between IFI16 and CHK2 or between IFI16 and γH2AX under any conditions (Fig 2D, 1^st^ and 2^nd^ rows, 5th and 6th blocks). In contrast, during KSHV infection, we observed significant increased nuclear and cytoplasmic interactions between IFI16 and BRCA1 (Fig 2D bar graph) as well as increased nuclear and cytoplasmic interactions between IFI16 and ASC (Fig 2D, 3^rd^ row, 1^st^ and 4^th^ blocks). In addition, we also observed only a limited association of BRCA1 with CHK2 and γH2AX (Fig 2D, 3^rd^ row, 2^nd^ and 3^rd^ blocks) and no overall interaction of IFI16 with CHK2 and γH2AX during infection (Fig 2D, 3^rd^ row, 5^th^ and 6^th^ blocks; S1 Table).

These observations suggested that: a) IFI16 interacts only with BRCA1 and not with H2AX and CHK2 under physiological conditions, b) the increase in IFI16-BRCA1 interaction observed in the infected cells was due to KSHV which is distinct from the complexes formed by BRCA1, H2AX and CHK2 proteins during DDR (S1 Table), and c) the BRCA1 and IFI16 complex may have roles during KSHV infection.

### *De novo* KSHV infection results in BRCA1 cytoplasmic distribution as part of the IFI16-ASC inflammasome complex

In response to KSHV infection, IFI16 interacts with the adaptor ASC, which recruits procaspase-1 to form an active inflammasome complex that gets relocated to the cytoplasm [2]. Since we detected increased association between BRCA1 and IFI16 in KSHV infected cells and observed increased IFI16-BRCA1 in the cytoplasm of infected cells (Fig 2D, 3^rd^ row, 1^st^ block), we next determined whether BRCA1 relocalizes to the cytoplasm in a way similar to that of IFI16 during *de novo* KSHV infection [2]. Although BRCA1 was observed in the nucleus and in the cytoplasm of both uninfected and infected cells, BRCA1 levels in the cytoplasm of infected cells increased during the observed periods (0.5 h, 4 h and 24 h) of infection similar to that of IFI16 (Fig 3A, panels 1 and 2, lanes 1 to 8). Forward and reverse co-IP experiments with the same uninfected and KSHV infected HMVEC-d nuclear lysates showed increased nuclear association between BRCA1 and IFI16 during the observed 0.5 h, 4 h and 24 h p.i. (Fig 3B). No such association was observed with IgG control (Fig 3B).

**Fig 3:** Cytoplasmic distribution of BRCA1 and IFI16 during *de novo* KSHV infection and BRCA1 is part of the IFI16 inflammasome complex. **(A)** Nuclear and cytoplasmic extracts from uninfected and KSHV infected HMVEC-d cells were western blotted (WB) with anti-BRCA1 and anti-IFI16 antibodies. Fraction purity and equal loading were assessed by western blots (WBs) for TBP and tubulin. **(B)** Nuclear extracts from experiment A were IP-ed with anti-BRCA1,-IFI16 antibodies and WB for IFI16 and BRCA1 respectively. Respective inputs were assessed by WB. Species specific IgG antibodies were used for specificity controls. **(C)** Cytoplasmic extracts from experiment A were IP-ed with anti-BRCA1,-IFI16,-Caspase1 or-ASC antibodies and WB for BRCA1, IFI16 and Caspase-1. Species specific IgG antibodies were used for specificity controls. Equal immunoprecipitation inputs were assessed by BRCA1, IFI16, ASC, Caspase-1, Tubulin and TBP WBs.

To determine whether BRCA1 was in complex with IFI16 in the cytoplasm of infected cells, cytoplasmic fractions were IP-ed with anti-BRCA1 antibodies and Western blotted for IFI16 (Fig 3C, panel 1). IFI16 was detected in the BRCA1 immunoprecipitates only in the cytoplasmic fractions of infected cells. In addition, we observed that the IFI16-BRCA1 interactions increased significantly with the duration of infection (Fig 3C, panel 1, lanes 3 to 5 vs lane 2). This observation was further confirmed by performing reverse-IP with anti-IFI16 antibodies and western blotting for BRCA1 (Fig 3C, panel 2, lanes 3 to 5 vs. lane 2).

Next, we determined whether the cytoplasmic BRCA1 was part of the active IFI16 inflammasome complex that gets relocalized to the cytoplasm during KSHV infection. Cytoplasmic fractions were IP-ed with anti-ASC, anti-IFI16, anti-BRCA1 and anti-procaspase-1 antibodies and Western blotted for IFI16, BRCA1 and procaspase-1 (Fig 3C, panels 3 to 9). Infection induced IFI16-inflammasomes were shown by the increased detection of IFI16 and cleaved Caspase-1 in the cytoplasm. The purity of the cytoplasmic preparation was confirmed by the absence of TBP and the presence of tubulin (Fig 3C, bottom input panels). Cytoplasmic relocalization of the active IFI16 inflammasome complex during KSHV infection was observed by the progressively increased interactions between ASC, IFI16 and procaspase-1 (Fig 3C, panels 3, 5, 7 and 9, lanes 3 to 5 vs lane 2). We also observed the presence of increasing amounts of BRCA1 in ASC and procaspase-1 immunoprecipitates during the course of infection (Fig 3C, panels 4 and 8, lanes 3 to 5 vs. lane 2). These observations for the first time identified the previously unknown association of BRCA1 with ASC and procaspase-1. Immunoprecipitation of procaspase-1 by anti-BRCA1 antibodies (Fig 3C, panel 6, lanes 3 to 5 vs. lane 2) suggested that BRCA1 relocated to the cytoplasm during KSHV infection as a component of the active IFI16 inflammasome complex.

Fig 3A showing KSHV infection induced cytoplasmic distribution of a fraction of nuclear resident BRCA1 and IFI16 coupled with the observed increase in co-IP of BRCA1 and IFI16 in the nuclear as well as the cytoplasmic fractions during virus infection (Fig 3B and 3C) suggest that BRCA1-IFI16 association in the nucleus increase perhaps to sense the viral genome which is followed by the BRCA1 aided cytoplasmic translocation of IFI16.

### PLA studies confirm that *de novo* KSHV infection results in BRCA1 cytoplasmic distribution as part of the IFI16-ASC inflammasome complex

To further confirm the association of IFI16, ASC and procaspase-1 with BRCA1, we performed PLA in uninfected HMVEC-d cells and cells infected with KSHV for 24 h using anti-IFI16, anti-BRCA1, anti-ASC and anti-procaspase-1 antibodies. Specificity of the assay was confirmed by using secondary antibodies linked to probes alone (Fig 4B) and also by using only one primary antibody plus both secondary antibodies linked to probes (S2 Fig, A to E). The lack of detection of any signal following PLA in all cases confirmed the specificity of all the antibodies tested (Fig 4B and S2 Fig, A to E). When we used rabbit and mouse anti-IFI16 antibodies against different IFI16 epitopes in PLA for detecting cellular localization of IFI16 during infection, we detected IFI16 in the nucleus of uninfected cells (Fig 4A, UI, red arrows). In contrast, as we have demonstrated previously [3], at 24 h p.i., IFI16 was detected in both the nucleus and the cytoplasm of infected cells (Fig 4A, KSHV 24 h, red and yellow arrows).

**Fig 4:** PLA and knockdown studies demonstrating specificity of BRCA1 interactions with IFI16-inflammasome components and relocalization to the cytoplasm during *de novo* KSHV infection. **(A)** PLA detecting IFI16 in uninfected and KSHV infected HMVEC-d cells. Red dots are indicative of PLA reactions representing the subcellular distribution of IFI16. Red arrows: nuclear IFI16. Yellow arrows: cytoplasmic IFI16. (**B**) Specificity control for PLA using only secondary antibodies. **(C-G)** PLA (red dots) detecting various complexes in uninfected (left panels) and *de novo* KSHV infected HMVEC-d cells at 24 h p.i. (right panels). Red arrows: nuclear PLA. Yellow arrows: cytoplasmic PLA. (C) IFI16 and BRCA1 complexes. (D) IFI16 and ASC complexes. (E) BRCA1 and ASC complexes. (F) BRCA1 and caspase-1 complexes. (G) IFI16 and Caspase-1 complexes. Boxed areas are enlarged. Quantitative analysis of the average number of PLA spots per cell and that of nucleus vs cytoplasm of infected cells is presented in the rightmost columns. ***: p<0.001, **: p<0.01, and ns: not-significant. **(H)** Effect of IFI16 knockdown on BRCA1-ASC association during KSHV infection. HMVEC-d cells treated with control Si-RNA (Si C) or IFI16-Si-RNA (Si IFI16) were infected with KSHV and lysates were IP-ed with anti-BRCA1 antibodies followed by WB with anti-ASC antibodies. Blots were stripped and probed with anti-BRCA1 antibodies to detect the presence of BRCA1. WCLs were used as input controls for WBs to show IFI16 knockdown, presence of ASC and cleavage of procaspase-1. **(I)** BRCA1 does not interact with AIM2 and NLRP3. Uninfected or KSHV infected HMVEC-d cell lysates were IP-ed with anti-BRCA1 antibodies followed by WB with anti-NLRP3 or AIM2 antibodies. Equal inputs for IPs were assessed by NLRP3, AIM2 and BRCA1 WBs. β-actin was used as an equal loading control. HC and LC: IgG heavy and light chains, respectively.

To assess the associations with inflammasome related proteins, next, we performed PLA in uninfected and KSHV infected HMVEC-d cells at 24 h p.i. using various combinations of anti-IFI16 and anti-BRCA1 antibodies. We observed that, compared to uninfected cells, in addition to nuclear IFI16-BRCA1 interactions (Fig 4C, UI versus KSHV 24 h, red arrows), a substantial amount of BRCA1 and IFI16 were detected in the cytoplasm of infected cells (Fig 4C, yellow arrows and bar graph). PLA performed to determine the interactions of BRCA1, IFI16 and ASC in infected and uninfected HMVEC-d cells (Fig 4D to 4G) showed increased interactions between IFI16 and ASC (Fig 4D, red and yellow arrows), BRCA1 and ASC (Fig 4E, red and yellow arrows), BRCA1 and procaspase-1 (Fig 4F, red and yellow arrows) and IFI16 and procaspase-1 (Fig 4G, red and yellow arrows) in the cytoplasm of infected cells at 24 h p.i. compared to the uninfected cells as indicated by the detection of a significantly higher number of PLA spots (respective bar graphs). However, comparison between the number of BRCA1 and IFI16 PLA spots as well as IFI16 and ASC PLA spots detected in the infected cell nucleus and cytoplasm were not significant (Fig 4C and 4D, respective bar graphs) which could be due to complex formation as a result of continuous and dynamic viral genome sensing events and/or formation of different molecular complexes with distinct functionality. In contrast, PLA analysis showed that there were significant increases in the association of IFI16 with Caspase-1 as well as BRCA1 with ASC and Caspase-1 in the cytoplasm of infected cells compared to the nucleus of infected cells (Fig 4E–4G, respective bar graphs) which probably represent the active inflammasome complex in the cytoplasm.

These observations confirmed that BRCA1 interacts with components of the IFI16 inflammasome complex and relocalizes to the cytoplasm during *de novo* KSHV infection.

### KSHV infection induced association of BRCA1 with inflammasome adaptor ASC is dependent on IFI16

Although BRCA1 lacks a PYD domain to interact directly with the PYD domain of ASC, the similarities of the BRCA1 association with ASC to that of IFI16 with ASC prompted us to investigate whether the BRCA1-ASC interaction requires the presence of IFI16. Therefore, we analyzed the effect of IFI16 knockdown on the ASC-BRCA1 association early during KSHV infection (4 h) in HMVEC-d cells. Compared to control Si-RNA, >90% of IFI16 was knocked down with Si-IFI16 RNA (Fig 4H, panel 3, lanes 2 and 4 vs. lanes 1 and 3). Specificity of IFI16 knockdown was shown by the absence of any overall changes in the expression of BRCA1 and ASC protein levels (Fig 4H).

Cell lysates from control or IFI16-Si-RNA transfected HMVEC-d cells either uninfected or infected with KSHV were used for IP with BRCA1 antibody followed by Western blot with ASC antibodies. While the uninfected cells showed very little or no association of ASC with BRCA1 (Fig 4H, panel 1, lane 1–2), ASC was found in BRCA1 immunoprecipitates from control Si-RNA treated KSHV infected cells (Fig 4H, panel 1, lane 3). In contrast, little or no ASC was co-IP-ed with BRCA1 in Si-IFI16 treated virus infected cells (Fig 4H, panel 1, lane 4). There were no overall changes in the IP-ed total BRCA1 (Fig 4H, panel 2) or in total ASC and β-actin levels (Fig 4H, panels 5 and 6), which demonstrated the specificity of the IFI16 knockdown with few off-target effects. The presence of cleaved Caspase-1 in control Si-RNA treated KSHV infected cells but not in uninfected cells and little or none in Si-IFI16 treated virus infected cells (Fig 4H, panel 4) confirmed the activation of the IFI16 inflammasome during KSHV infection [2] and specificity of the experiment.

Next, we analyzed the BRCA1 cellular distribution by PLA in IFI16 knockdown HMVEC-d cells infected with KSHV (4 h p.i.) (S3A and S3B Fig). As shown before, IFI16 PLA spots were detected in the nucleus and in the cytoplasm of infected cells which were significantly absent in the Si-IFI16 cells and the efficiency of IFI16 knockdown is shown by the significant >95% reduction of IFI16 PLA spots (S3A Fig and bar graph). We observed that compared to uninfected Si-control cells with some amount of BRCA1 in the cytoplasm, KSHV infection resulted in increased BRCA1 cytoplasmic distribution which was significantly less in the IFI16 knockdown virus infected cells with a level comparable to that of the uninfected cells (S3B Fig and bar graph).

These results suggested that KSHV induced association of BRCA1 (with no PYD domain) with inflammasome adaptor ASC (with PYD domain) relies on the presence of IFI16 with PYD domain, and demonstrated the dependence on IFI16 for the observed BRCA1–ASC association and increased cytoplasmic BRCA1 translocation during KSHV infection.

### KSHV infection does not induce the association of BRCA1 with cytoplasmic inflammasome NLRP3 and AIM2 sensors

To determine whether BRCA1 is a general inflammasome component or is specific only for the IFI16 inflammasome, protein lysates from HMVEC-d cells infected with KSHV for 4 h (early) and 24 h (late) were IP-ed with anti-BRCA1 antibodies and Western blotted for NLRP3 and AIM2 proteins. As shown in Fig 4I, panels 1 and 2, NLRP3 and AIM2 were not associated with BRCA1 in the uninfected or infected cells. No significant changes in the total protein levels of BRCA1, NLRP3 and AIM2 were observed (Fig 4I, input panels). These results not only demonstrated the specific interaction of BRCA1 with IFI16 but also ruled out its association with other cytoplasmic inflammasome sensors under physiological conditions as well as during KSHV infection.

### Latent KSHV infection enhances the IFI16 and BRCA1 interaction, their association with adaptor ASC, interaction of Caspase-1 with ASC and BRCA1, and induces their cytoplasmic distribution

Primary Effusion Lymphoma (PEL) derived BCBL-1 cells are KSHV latently infected B-cells with >80 copies of nuclear KSHV genomes and we have shown previously that IFI16 colocalizes with nuclear KSHV genome in latently infected cells resulting in the constitutive activation of IFI16 inflammasomes [3]. To examine the IFI16-BRCA1 interaction and redistribution in cells latently infected with KSHV, we used a combination of IP reactions with anti-IFI16,-BRCA1 or-ASC antibodies and Western blot reactions with cytoplasmic fractions from latent KSHV positive BCBL-1 and TIVE-LTC (endothelial) cells (Fig 5A and 5B) and also *de novo* KSHV infected (24 h) human foreskin fibroblast (HFF) cells (S4A Fig). We observed the association of BRCA1 with IFI16, ASC and Caspase-1 in the cytoplasm of infected cells (Fig 5A and 5B and S4A Fig) but not in the cytoplasmic fractions of control KSHV negative BJAB and TIVE (endothelial) (Fig 5C and 5D) or uninfected HFF cells.

**Fig 5:** Analysis demonstrating BRCA1 is a member of the IFI16-inflammasome complex in cells latently infected with KSHV. **(A-D)** Cytoplasmic fractions of KSHV latently infected B lymphoma BCBL-1 (A) and endothelial TIVE-LTC (B) cells, and KSHV-negative B lymphoma BJAB (C) and endothelial TIVE (D) cells were IP-ed with anti-IFI16, BRCA1 or ASC antibodies and western blotted for IFI16, BRCA1 and caspase-1. IgG antibodies were used for specificity controls. Equal inputs for IPs were assessed by BRCA1, IFI16, ASC and Caspase-1 WBs, while tubulin and TBP WBs were done to confirm purity of cytoplasmic fractions. **(E-I)** PLA detecting IFI16 and BRCA1 complexes (E), IFI16 and ASC complexes (F), BRCA1 and ASC complexes (G), ASC and Caspase-1 complexes (H) and BRCA1 and Caspase-1 complexes (I) in KSHV-negative TIVE and KSHV positive TIVE-LTC cells. Boxed areas are enlarged. Red dots represent IFI16-BRCA1, IFI16-ASC, BRCA1-ASC, ASC-Caspase-1 or BRCA1-Caspase-1 complexes. Yellow arrows indicate cytoplasmic localization of IFI16-BRCA1, IFI16-ASC, BRCA1-ASC, ASC-Caspase-1 or BRCA1-Caspase-1 complexes. Red arrows indicate nuclear localization of IFI16-BRCA1, IFI16-ASC or BRCA1-ASC, ASC-Caspase-1 or BRCA1-Caspase-1. Quantitative analysis of the average number of PLA spots/cell and that of nucleus vs cytoplasm of infected cells is presented in the right most columns. *: p<0.05; ***: p<0.001 and ns: not significant.

These observations were further validated by PLA. Compared to TIVE cells (Fig 5E to 5I, left panels), we observed increased interactions between IFI16-BRCA1, IFI16-ASC, BRCA1-ASC, ASC-Caspase1 and BRCA1-Caspase1, and their distribution in the cytoplasm of KSHV latent TIVE-LTC cells (Fig 5E to 5I, right panels, yellow arrows, graphs in rightmost column). Analysis of average PLA spots showed a significant increase in the association of ASC with Caspase-1 (Fig 5H, graphs in rightmost column) as well as BRCA1 with ASC and Caspase-1 (Fig 5G and 5I, graphs in rightmost column) in the cytoplasm compared to nucleus of virus infected cells as observed before.

Similarly, using PLA, we also observed increased interactions and cytoplasmic distribution of IFI16-BRCA1 and IFI16-ASC complexes in HFF cells infected with KSHV for 24 h (S4B and S4C Fig, lower panels, yellow arrows).

Together with the biochemical studies, these PLA studies strongly demonstrated that KSHV latent infection also induced the association of nuclear sensor IFI16 with BRCA1 to interact with ASC and Caspase-1 and their redistribution to the cytoplasm of infected cells.

### The increase in the BRCA1-IFI16 and IFI16-ASC associations and their cytoplasmic distribution occurs in cells containing nuclear herpesviral genome but not during vaccinia virus infection

Similar to the biochemical studies with B cells and TIVE-LTC cells latently infected with KSHV described above, PLA studies also validated the increased interactions between IFI16-BRCA1, IFI16-ASC, and BRCA1-ASC and their distribution in the cytoplasm of KSHV positive BCBL-1 cells (Fig 6A to 6C, right panels, white arrows) compared to KSHV negative BJAB cells (Fig 6A to 6C, left panels). These results demonstrated that BRCA1 is part of the IFI16 inflammasome complex in B cells with latent nuclear KSHV genome.

**Fig 6:** Analysis demonstrating that infection by nuclear DNA virus is essential for IFI16, ASC, BRCA1 and Caspase-1 associations and for BRCA1 association with IFI16 inflammasome components. **(A-C)** PLA detecting IFI16 and BRCA1 complexes (A), IFI16 and ASC complexes (B) and BRCA1 and ASC complexes (C) in KSHV-negative BJAB and KSHV positive BCBL-1 cells. Arrows indicate cytoplasmic localization of complexes. **(D and E)** PLA detection of IFI16-ASC (D) and BRCA1-IFI16 (E) interactions in EBV positive and negative B-cells. Red spots indicate PLA signals. Arrows indicate IFI16-ASC complexes and IFI16-BRCA1 complexes in the cytoplasm of EBV positive LCL cells. **(F and G)** PLA detection (red spots) of IFI16-BRCA1 (upper panels), BRCA1-ASC (middle panels) and BRCA1-Caspase-1 (bottom panels) in PBMC following 4 h p.i. with KSHV or EBV. Arrows indicate cytoplasmic localization of complexes. **(H and I)** PLA detection of AIM2-ASC (yellow arrows), IFI16-ASC and IFI16-BRCA1 (white arrows) complexes in uninfected (H) and vaccinia virus infected HMVEC-d cells (8 h p.i.) (I).

Our previous studies demonstrated the constitutive activation of IFI16 inflammasomes in EBV infected cells as well as the colocalization of nuclear IFI16 with the nuclear EBV genomes [4]. In contrast, in cells infected with vaccinia virus replicating its dsDNA in the cytoplasm of infected cells, we observed the activation of the cytoplasmic AIM2-ASC inflammasome and not the IFI16-ASC inflammasome [2]. To determine whether BRCA1 and IFI16 interactions also occur in EBV infected cells, we performed PLA in cells infected with EBV and vaccinia virus. As expected, we observed a significantly increased interaction between IFI16 and ASC, and their distribution in the cytoplasm in EBV latency III positive lymphoblastoid cells (LCL) compared to control EBV negative B-lymphoma Akata and Ramos cells (Fig 6D, panels 1 and 2 versus panel 3, yellow arrows). Furthermore, we also observed increased interactions between IFI16 and BRCA1 and their cytoplasmic distribution in EBV positive cells compared to Ramos and Akata cells (Fig 6E, panels 3 vs panels 1and 2, yellow arrows). *De novo* KSHV or EBV infection (4 h p.i.) in PBMC also showed IFI16-BRCA1, BRCA1-ASC and BRCA1-Caspase-complex formation and their cytoplasmic distribution as observed by PLA (Fig 6F and 6G).

In contrast to the nuclear replicating herpesvirus infected cells, compared to uninfected cells, we observed very high association of ASC and AIM2 in the cytoplasm of vaccinia infected cells (Fig 6H versus Fig 6I, panel 1) and very little or no interaction between IFI16 and ASC (Fig 6H versus Fig 6I, panel 2). More importantly, we did not observe any significant increase in the IFI16-BRCA1 interactions in vaccinia infected cells compared with uninfected cells (Fig 6H versus Fig 6I, panel 3). These results demonstrated the specificity of BRCA1-IFI16 interactions observed in KSHV and EBV infected cells and suggest that the presence of nuclear viral DNA is necessary for increased BRCA1-IFI16 interactions, association with ASC and their cytoplasmic redistribution.

### BRCA1 is part of the same IFI16-ASC complex formed as a response to nuclear KSHV and EBV genomes

We next determined whether BRCA1, IFI16 and ASC are in a single macromolecular complex in cells latently infected with KSHV. For this, we performed double sequential PLAs with an initial reaction for IFI16 and BRCA1 (Fig 7A–7D, red spots) followed by a reaction for IFI16 and ASC (Fig 7A–7D, green spots). Very low numbers of green and red PLA spots, mostly distinct, were detected predominantly in the nucleus of KSHV negative BJAB and EBV negative Ramos cells (Fig 7A and 7C). In contrast, significantly higher red and green PLA spots with a higher number of colocalizing yellow spots were observed in KSHV positive BCBL-1 and EBV positive LCL cells (Fig 7B and 7D, white arrow). Interestingly, some white PLA colocalization spots were also detected in the nuclei of BCBL-1 cells (Fig 7B); however, yellow spots were mainly distributed in the cytoplasmic region. These results showed that IFI16, BRCA1 and ASC were in close proximity, suggesting the formation of an individual macromolecular complex, thus corroborating the results presented above. In addition, these results clearly demonstrated that the presence of nuclear viral genomes is critical for the formation of the innate BRCA1-IFI16-ASC inflammasome complexes.

**Fig 7:** Analysis demonstrating that IFI16, ASC and BRCA1 are present in the same molecular complex in KSHV and EBV infected cells. **(A and D)** Double sequential PLA of IFI16-BRCA1 and IFI16-ASC complexes. The PLA for IFI16 and BRCA1 was performed first using rabbit anti-IFI16 and mouse anti-BRCA1 antibodies and detected by DUOLink red detection agent. Cells were then washed, blocked with PLA reaction buffer and subjected to a second PLA reaction using mouse anti-IFI16 and goat anti-ASC antibodies and detected with DUOLink green detection agent. Nuclei were stained with DAPI (blue). Boxed areas are enlarged. Arrows indicates cytoplasmic colocalization (yellow spots) of red PLA signals (representing IFI16-BRCA1 complexes) or green PLA signals (representing IFI16-ASC complexes) in BCBL-1 (KSHV +ve) (B) and LCL (EBV +ve) (D) vs BJAB (KSHV-ve) (A) and Ramos (EBV-ve) cells (C).

### BRCA1 is necessary for IFI16 inflammasome activation and its cytoplasmic relocalization

The association of BRCA1-IFI16 with ASC and Caspase-1 prompted us to determine the functional role of BRCA1 in the regulation of IFI16-inflammasome formation leading to cleavage of procaspase-1 into active Caspase-1 followed by cleavage of pro-IL-1β into functional IL-1β.

To assess the role of BRCA1, we performed BRCA1 knockdown using a pool of Si-RNAs against BRCA1 (Si-BRCA1). The uninfected and KSHV infected Si-Control and Si-BRCA1 HMVEC-d and HFF cells (at 0.5 h, 4 h and 24 h p.i.) were used for biochemical studies to determine the effects of BRCA1 knockdown on the cleavage of procaspase-1 and/or pro-IL-1β. Specificity of BRCA1 knockdown was shown by the absence of any overall changes in the expression of IFI16 and ASC protein levels (Fig 8). These results demonstrated that although BRCA1-IFI16 are functionally related to each other, the expression level of these proteins are independent of their functionality.

**Fig 8:** Analysis demonstrating that BRCA1 is essential for IFI16 inflammasome activation. **(A-D)**. Control Si-RNA (Si-Cont) treated and BRCA1 (Si-BRCA1) knockdown HMVEC-d cells (A), HFF cells (B), BRCA1 positive (+) 184B5 and negative (-) HCC1937 breast tumor epithelial cell lines (C) and BRCA1 (-) HCC1937 cells transduced with lentivirus encoding human BRCA1 (D) were infected with KSHV for the indicated times. Lysates were analyzed by WBs to detect BRCA1, cleaved IL-1β (p17), Caspase-1 (p20), IFI16 and ASC. β-actin was used as an equal loading control. Lysates were also IP-ed with anti-ASC antibodies and western blotted to detect IFI16 and procaspase-1.

Compared to Si-Control, >90% of BRCA1 knockdown was observed in Si-BRCA1 cells (Fig 8A and 8B, panel 1, lanes 1–5 vs lanes 6–8). Cleaved Caspase-1 (p20) and cleaved, mature IL-1β (p17) was detected in KSHV infected Si-Control HMVEC-d cells (Fig 8A, panels 2 and 3, lanes 3–5). Similarly, the presence of mature IL-1β was observed only in KSHV infected Si-Control HFF cells (Fig 8B, panel 2, lanes 3–5). However, no detectable cleavage of Caspase-1 and/or IL-1β was observed in Si-BRCA1 treated KSHV infected cells at any time of infection (Fig 8A, panels 2 and 3, lanes 6–8 and Fig 8B, panel 2, lanes 6–8). Additionally, we did not observe any marked changes in the expression levels of IFI16, ASC or β-actin as a result of BRCA1 knockdown (Fig 8A, panels 4, 5 and 8 and Fig 8B, panels 3,4 and 7), indicating the specificity of knockdown and the absence of off-target effects due to BRCA1 knockdown.

To further determine the role of BRCA1 in KSHV infection-induced inflammasome activation, we utilized a human mammary epithelial cell line with wild type BRCA1 (184B5 BRCA1^+^) and with a BRCA1 null mutant (HCC1937, BRCA1^–^) [20] (Fig 8C panel 1). Similar to BRCA1 knockdown in HMVEC-d and HFF cells, significant levels of active Caspase-1 (p20) and mature IL-1β (p17) were observed in BRCA1^+^ cells both at early (0.5 h and 4 h) as well as late (24 h) times p.i. but not in BRCA1^–^ cells (Fig 8C, panels 2 and 3, lanes 2–4 vs. lanes 6–8) or in uninfected cells (Fig 8C, panels 2 and 3, lane 1 vs lane 5). To further confirm the active involvement of BRCA1 in KSHV induced inflammasome activation, we transduced BRCA1^–^ HCC cells with lentiviruses expressing BRCA1 (Fig 8D, panel 1, lanes 5–8) or control lentiviruses (Fig 8D, panel 1, lanes 1–4). As expected, cleaved Caspase-1 and mature IL-1β were observed in BRCA1 expressing but not in BRCA1 negative HCC 1937 cells during either the early or late period post-KSHV infection (Fig 8D, panel 2 and 3, lanes 6–8 vs lanes 1–5). Together, these results demonstrated the active participation of BRCA1 in the formation of functionally active Caspase-1 and mature IL-1β during KSHV infection.

We next determined the potential molecular mechanism responsible for the observed dramatic reduction in inflammasome activation due to BRCA1 knockdown or absence. Since IFI16 inflammasome activation needs simultaneous interaction of adaptor ASC with both IFI16 and procaspase-1, we investigated the physical associations among IFI16 inflammasome components (IFI16, ASC, Caspase-1) in the BRCA1 knockdown cells, in the absence of functional BRCA1 or in lenti-BRCA1 add- back to BRCA1 negative cells. Cell lysates from control or BRCA1-Si-RNA-transfected HMVEC-d or HFF cells either uninfected or infected with KSHV were used for IP with anti-ASC antibody followed by WB with anti-IFI16 or Caspase-1 antibodies. While the uninfected cells showed very little or no association of ASC with IFI16 and Caspase-1, these associations were prominently observed in ASC immunoprecipitates of Si-Control treated KSHV infected cells both at early (0.5 and 4 h) as well as late (24 h) times p.i. (Fig 8A, panels 6–7 and Fig 8B, panels 5–6, lanes 3–5 vs lanes 1–2). In contrast, little or no IFI16 or Caspase-1 was co-IP-ed with ASC in Si-BRCA1 treated virus infected cells (Fig 8A, panels 6–7 and Fig 7B, panels 5–6, lanes 6–8).

Furthermore, we observed the presence of IFI16 and Caspase-1 in ASC immunoprecipitates predominantly in KSHV infected BRCA1 ^+^ 184B5 cells but not in BRCA1 ^−^HCC1937 cells (Fig 8C, panel 6–7, lanes 2–4 vs lane 1 and 5 and lanes 6–8) as well as in lenti-BRCA1 expressed but not in control lenti-vector transduced HCC1937 cells upon early and late KSHV infection over uninfected cells (Fig 8D, panels 5–6, lane 6–8 vs lanes 1–5). However, there were no marked changes in the expression of IFI16, ASC and β-actin in any of these conditions.

We further analyzed the effect of BRCA1 knockdown on IFI16-ASC interactions by PLA during *de novo* KSHV infection in HMVEC-d and HFF cells. Although a considerable amount of IFI16 was detected in the nucleus of both uninfected and KSHV infected Si-Control and si-BRCA1 HMVEC-d cells (Fig 9A and 9B), cytoplasmic redistribution of IFI16 molecules was predominantly observed in Si-Control cells compared with that in Si-BRCA1 cells (Fig 9A vs. Fig 9B, yellow arrows). Next, we assessed the IFI16-ASC interactions in uninfected and KSHV infected Si-Control and si-BRCA1 HMVEC-d and HFF cells. Compared to uninfected HMVEC-d and HFF cells, we observed more IFI16-ASC PLA spots, indicating increased interactions in Si-Control cells at both early and late times post-KSHV infection (Figs 9C and 8E vs Fig 9D and 9F). In addition, considerable numbers of the observed PLA spots were redistributed to the cytoplasm after 4 h and 24 h of infection (Fig 9C, white arrows and Fig 9E, yellow arrows). In contrast, in Si-BRCA1 cells, very few IFI16 and ASC PLA spots were seen at either early or late times post-KSHV infection, implying very few interactions (Fig 9D and 9F). These findings suggested that BRCA1 is essential for IFI16-ASC complex formation and its cytoplasmic translocation during *de novo* KSHV infection.

**Fig 9:** PLA analysis demonstrating the importance of BRCA1 for IFI16 and ASC complex formation and redistribution of IFI16 and IFI16-ASC complex during KSHV infection. **(A)** Control Si-RNA (Si-control) treated and **(B)** BRCA1 (Si-BRCA1) knockdown HMVEC-d cells were infected with KSHV (30 DNA copies/cell) for 30 min, 4 h and 24 h. Cells were subjected to PLA reactions using mouse and goat anti-IFI16 antibodies, washed and then reacted with species specific secondary antibodies linked with PLA probes. PLA reactions were detected using DUOLink red detection agent. Red dots indicate IFI16 and yellow arrows indicate cytoplasmic localization of IFI16 at the indicated time periods. IFI16 and ASC association during *de novo* KSHV infection in BRCA1 knockdown HMVEC-d **(C and D)** and HFF **(E and F)** cells. Control Si-RNA (Si-Cont) (C and E) treated and BRCA1 (Si-BRCA1) (D and F) knockdown cells were infected with KSHV for the indicated times. Red dots indicate IFI16-ASC complexes. Arrows indicate cytoplasmic IFI16-ASC complexes.

Collectively, these results clearly demonstrated the essential role of BRCA1 in regulating KSHV induced IFI16 cytoplasmic redistribution and assembly of the IFI16-ASC-Caspase-1 inflammasome complex and IFI16 inflammasome activation.

### BRCA1 promotes KSHV genome recognition by IFI16 and correlates with activation of the inflammasome response mediated by IFI16

IFI16 acts as a nuclear DNA sensor for KSHV, EBV and HSV-1 genomes and induces inflammasome activation [2, 4, 5]. It also recruits the endoplasmic resident protein STING to interact with TBK1 and IRF3, leading to phosphorylation and nuclear translocation of IRF3 in herpes virus infected cells [6,7]. Based on our findings that (i) BRCA1 interacts with IFI16 and ASC, and undergoes cytoplasmic translocation as part of the IFI16 inflammasome complex during *de novo* and latent KSHV and EBV infections, (ii) the presence of nuclear herpes viral DNA is necessary for BRCA1-IFI16 and IFI16-ASC interactions and, (iii) the absence of BRCA1 impaired IFI16 cytoplasmic translocation, IFI16-ASC-Caspase-1 associations and IFI16 inflammasome activation, we hypothesized that although IFI16 can directly bind to DNA in artificial systems [1], in the dynamic nuclear environment during herpes virus infections, BRCA1 is necessary for recognizing nuclear viral DNA by IFI16. This phenomenon results in cytoplasmic translocation of IFI16, activation of IFI16 inflammasomes and induction of host innate responses such as type-I interferon production.

To test this, we determined whether the BRCA1-IFI16 complex recognizes the KSHV genome by infecting HMVEC-d and HFF cells for 24 h with KSHV containing 5-ethynyl-2’-deoxyuridine (EdU) labeled viral genomes (Fig 10A and 10B, panels 1, 3 and 4, red spots within DAPI stained nuclei) and performed PLA for IFI16-BRCA1. In the combined PLA-IFA images, many of the IFI16-BRCA1 (green) complexes colocalized with KSHV genomes (red) in the nuclei (Fig 10A and 10B, yellow spots (BRCA1-IFI16+EdU) in panel 2 and white spots (BRCA1-IFI16+EdU+DAPI) in panel 3 and the yellow arrows of enlarged images in panel 4), which demonstrated possible viral genome sensing events mediated by this complex. A considerable number of BRCA1-IFI16 complex green spots were observed in the cytoplasm in addition to those in infected cell nuclei (Fig 10A and 10B, panels 2–4, red arrows) implying a virus dependent translocation of IFI16-BRCA1 complexes as demonstrated in our results described earlier.

**Fig 10:** Analysis demonstrating that BRCA1 is involved in the recognition of KSHV genomes by IFI16. **(A and B)** HMVEC-d cells (A) and HFF cells (B) were infected with EdU labeled KSHV for 24 h and IFI16-BRCA1 complexes were assessed by PLA. Nuclei were stained with DAPI and EdU labeled viral genomes detected by Click-reaction with Alexa 594 labeled azide. Boxed areas of merged images (PLA IFI16+BRCA1+DAPI+EdU labeled KSHV) are enlarged. Green PLA dots represent IFI16-BRCA1 complexes. Yellow arrows indicate colocalization of IFI16-BRCA1 complexes with EdU labeled KSHV genome. Red arrows indicate cytoplasmic localization of IFI16-BRCA1 complexes. **(C)** PLA demonstrating BRCA1 is a member of the IFI16 inflammasome and present in the same IFI16-ASC-BRCA1 complex during *de novo* KSHV infection. HMVEC-d cells were infected with EdU labeled KSHV (red) for 24 h. EdU labeled viral genomes were detected by Click-reaction with Alexa 594 labeled azide. Double sequential PLA was performed for colocalization of IFI16-BRCA1 and IFI16-ASC complexes. PLA reactions for IFI16 and BRCA1 were performed first using rabbit-IFI16 and mouse anti-BRCA1 antibodies (red). A second PLA reaction for IFI16 and ASC was performed using mouse anti-IFI16 and goat anti-ASC antibodies (green). Nuclei (DAPI-blue). Red EdU spots were also represented as blue spots in the bottom panels. White arrows: cytoplasmic colocalization (yellow spots) of PLA red (IFI16-BRCA1) and green (IFI16-ASC) signals. Orange arrows: white spots representing EdU genome colocalization with red IFI16-BRCA1 and green IFI16-ASC signals. **(D and E)** Absence of IFI16 association with KSHV genome in BRCA1 knockdown cells. Control Si-RNA (Si-Control) (D) and BRCA1 (Si-BRCA1) (E) knockdown HMVEC-d cells were infected with EdU labeled KSHV for 24 h. IFI16 was detected by PLA using mouse and goat anti-IFI16 antibodies. EdU labeled viral genomes were detected by Click-reaction with Alexa 594 labeled azide. Green PLA reaction dots indicate subcellular distribution of IFI16. Red arrows indicate cytoplasmic IFI16. Boxed areas of merged images are enlarged. White arrows (yellow spots) indicate association of IFI16 (PLA green dots) with EdU labeled KSHV genome (red).

To further demonstrate that the presence of nuclear KSHV genome drives the formation of BRCA1, IFI16 and ASC single macromolecular complexes, a sequential PLA with IFI16-BRCA1 and then IFI16-ASC was performed in HMVEC-d cells infected with EdU KSHV for 24 h. Red EdU spots within the nucleus demonstrated the infection and presence of viral genome (Fig 10C, panel 1) which were also represented as blue spots for the convenience of analysis (Fig 10C, panel 3 and 4). Considerable numbers of BRCA1-IFI16 red spots and IFI16-ASC green spots colocalized (yellow spots) in the nucleus as well as in the cytoplasm (white arrows). These results demonstrated the simultaneous presence of BRCA1-IFI16-ASC in a single complex. Most interesting was the detection of numerous white spots in the nucleus (Fig 10C, orange arrows) representing colocalization of BRCA1-IFI16 and IFI16-ASC complexes with the KSHV genome. These results demonstrated that the BRCA1-IFI16-ASC complexes recognize the presence of the foreign KSHV genome in the host cell nuclei.

Although some of the IFI16-ASC complexes (green spots) were also observed in very close proximity to the BRCA1-IFI16 complexes (red spots), distinct clear colocalization yellow spots were not visualized in all cases and some spots were distant from each other (Fig 10C). These might be due to the dynamic nature of one or more precomplexes followed by formation of mature inflammasome complexes that are >40 nm apart or formation of a complex with separate entities and distinct functionality.

To investigate the functional implications of BRCA1 in KSHV genome recognition by the BRCA1-IFI16 complex, we verified the consequence of BRCA1 knockdown affecting KSHV genome sensing by IFI16 in HMVEC-d cells at 24 h post-EdU KSHV infection. In control Si-RNA treated cells, we observed the colocalization of nuclear IFI16 molecules (green PLA spots) with EdU KSHV genome (red) (Fig 10D, panels 4 and 5, and Fig 11A, yellow spots, white arrows). As seen before, IFI16 was also detected in the cytoplasm without any colocalization with the viral genome probe (Fig 10D, panels 2, 3 and 4, green spots, red arrows and Fig 11A). These results demonstrated the cytoplasmic redistribution of IFI16 during KSHV infection and the absence of free viral genome in the cytoplasm. Multiple IFI16-DNA colocalization spots indicated interactions with several viral genomes in the presence of functional BRCA1. In contrast, IFI16 was confined to the nucleus of the BRCA1 Si-RNA treated cells with notably decreased colocalization with the EdU KSHV genome at 24 h p.i. (Fig 10E, panels 4 and 5 and Fig 11B and 11F). Consistent with this result, in contrast to Si-Control cells infected with KSHV, very little colocalization of IFI16 PLA spots and EdU KSHV genome was observed in BRCA1 knockdown HMVEC-d cells even at the early time of KSHV infection (Fig 11D and 11E vs Fig 11C). Taken together, these results convincingly demonstrated that in the dynamic nuclear environment, IFI16 relies on BRCA1 to increase its affinity to foreign KSHV DNA leading into stable inflammasome complex formation and translocation into the cytoplasm of infected cells.

**Fig 11:** PLA analysis demonstrating abrogation of KSHV genome recognition by IFI16 in the absence of BRCA1 during *de novo* infection. **(A and B)** Z-stack analysis of control Si-RNA (Si-control) and BRCA1 (Si-BRCA1) knockdown HMVEC-d cells infected with EdU labeled KSHV for 24 h. Images of ten 1μm thick Z planes were acquired and analyzed. EdU labeled KSHV genome was detected by reaction with Alexa 594 labeled picolylazide (red) and IFI16 was detected using PLA as described above. (A) The presence of a significant association of IFI16 with EdU labeled KSHV genome in Si-Control HMVEC-d cells (white arrows) is indicated by a yellow color in the XZ and YZ planes. (B) The absence of IFI16 association with EdU labeled KSHV genome in Si-BRCA1 HMVEC-d cells is shown by the absence of yellow spots (white arrows) in the XZ and YZ planes. **(C-F)** PLA analysis of the time course of KSHV *de novo* infection showing the effect of BRCA1 absence on KSHV genome recognition by IFI16. HMVEC-d cells with Si-Control or Si-BRCA1 (BRCA1 knockdown) were infected with EdU labeled KSHV for the indicated time periods. IFI16 was detected by PLA using mouse and goat anti-IFI16 antibodies (green). Nuclei were stained with DAPI. EdU labeled viral genome was detected using Alexa 594 labeled azide (red). Numbered boxed areas are enlarged and shown in the rightmost two panels. Green PLA reaction dots indicate IFI16. Arrows (yellow spots) indicate EdU labeled KSHV genome (red spots) and its association with IFI16 (PLA green dots).

### BRCA1 is necessary for the type-1 interferon responses mediated by IFI16 during *de novo* KSHV infection

To elaborate on the functional significance of BRCA1, we measured the bioactive form of IL-1β secreted as a consequence of inflammasome activation by KSHV infection. Compared to uninfected HMVEC-d cells, a significant but gradual increase in IL-1β secretion (~4.8–19 pg/ml) was observed from early to late times p.i. in control Si-RNA treated cells (Fig 12A). In contrast, treatment of BRCA1 Si-RNA resulted in dramatic reduction in IL-1β secretion (~1.6–3.2 pg/ml) (Fig 12A) which corroborated the active role of BRCA1.

**Fig 12:** Effect of BRCA1 knockdown on subsequent IFI16 dependent innate immune response activation during KSHV infection. **(A)** IL1-β levels determined by ELISA from cell culture supernatant of control Si-RNA (Si-Cont) treated or BRCA1 knockdown (Si-BRCA1) HMVEC-d cells either uninfected or infected with KSHV (30 DNA copies/cell) for the indicated times. Results presented are means ± SD (** p<0.01, *** p<0.001 from Si-Cont vs Si-BRCA1 cells with KSHV infection). (**B-F**) BRCA1 plays an important role in IFI16-dependent IFN-β induction upon KSHV infection. (B) HMVEC-d cells with Si-Control (left panel) or Si-BRCA1 (BRCA1 knockdown) (right panel) were infected with KSHV (30 DNA copies/cell) for 4, 8 and 24 h. Cells were subjected to PLA with anti-IFI16 and anti-STING. Green dots indicate IFI16 and STING interactions at the indicated time periods. Nuclei were stained with DAPI. (C) Western blot analysis showing pIRF3 and total IRF3 expression in control Si-RNA (Si-Cont) treated or BRCA1 (Si-BRCA1) knockdown HMVEC-d cells upon KSHV infection. (D) Western blot analysis showing phospho IRF3 and total IRF3 expression in BRCA1 (-) HCC1937 cells transduced (48 h) with lentivirus control or lentivirus encoding human BRCA1 and subsequently uninfected or KSHV infected for the indicated times. (E) IFA demonstrating phosphorylation and nuclear localization of IRF3 during *de novo* KSHV infection of control Si-RNA (Si-control) and BRCA1 (Si-BRCA1) knockdown HMVEC-d cells. HMVEC-d cells with Si-Control (left panel) or Si-BRCA1 (BRCA1 knockdown) (right panel) were infected with KSHV (30 DNA copies/cell) for 4 h, 8 h and 24 h. Cells were reacted with anti-phospho IRF3 antibodies, washed and then incubated with Alexa 488 (green) conjugated secondary antibodies. Nuclei were stained with DAPI (blue). pIRF3 is indicated by green spots. (F) Cell culture supernatant IFN-β levels determined by ELISA from control Si-RNA (Si-Cont) treated or BRCA1 knockdown (Si-BRCA1) HMVEC-d cells either uninfected or infected with KSHV for the indicated times. Results presented are means ± SD (n = 3; * p<0.05, ** p<0.01, *** p<0.001 from Si-Cont vs Si-BRCA1 cells with KSHV infection).

Because a fraction of IFI16-BRCA1 complexes did not colocalize with IFI16-ASC in our sequential PLA experiments (Figs 7B, 7D and 10C) and there was significant restriction in the IFI16 nuclear to cytoplasmic translocation by BRCA1 knockdown, we set out to determine the role of BRCA1 in IFI16 mediated type I interferon production. When we first investigated the association of IFI16-STING responsible for the initial signal cascade for IFN-β via PLA, compared to uninfected HMVEC-d cells, control Si-RNA treatment followed by KSHV infection resulted in increased association of IFI16-STING at 4 h and 8 h p.i. which decreased at 24 h p.i. In contrast, BRCA1 Si-RNA treatment resulted in a nearly complete abrogation of IFI16-STING PLA spots (Fig 12B, green PLA spots).

Next, we determined the downstream signal molecule pIRF3 levels by WB in BRCA1 knockdown or BRCA1 reintroduction to BRCA1 negative cells following KSHV infection. A gradual increase in the pIRF3 level was observed from 0.5 h p.i. which decreased somewhat at 24 h p.i. in Si-Control treated KSHV infected HMVEC-d cells (Fig 12C, upper panel, lanes 3–5 vs lanes 1–2). In contrast, there was a substantial decrease in pIRF3 levels in Si-BRCA1 treated cells at early as well as late times p.i. (Fig 12C, upper panel, lanes 6–8 vs lanes 3–5) with no apparent change in total IRF3 (Fig 12C, bottom panel).

Similarly, compared to uninfected and lenti-vector control transduced cells, lenti-BRCA1 expression in BRCA1 negative HCC1937 cells resulted in increased phosphorylation of IRF3 from 0.5 h p.i. which decreased somewhat at 24 h p.i. (Fig 12D, upper panel, lanes 6–8 vs lanes 2–4 and lanes 1 and 5) with no significant changes in total IRF3 levels (Fig 12D, bottom panel). Consistent with these findings, IFA studies also showed a significant increase in pIRF3 levels and translocation to the nucleus in control Si-RNA treated KSHV infected HMVEC-d cells up to 8 h p.i. and a decrease at 24 h p.i. (Fig 12E, 1^st^ and 2^nd^ rows). However, with BRCA1 knockdown, IRF3 phosphorylation and nuclear translocation was significantly reduced (Fig 12E, 3^rd^ and 4^th^ rows). When IFN-β release was measured by ELISA, compared to uninfected cells (~26 pg/ml), we observed a gradual increase of IFN-β secretion (~42 pg/ml, ~74 pg/ml, ~125 pg/ml, ~67 pg/ml, ~61 pg/ml at 0.5, 4, 8, 18 and 24 h p.i., respectively) in Si-Control treated KSHV infected cells. In contrast, in BRCA1 depleted KSHV infected cells, we observed a significant reduction in IFN-β secretion (Fig 12F).

Together, these results clearly highlighted the essential role of BRCA1 in the regulation of KSHV genome recognition by IFI16 and correlated with the subsequent IFI16 mediated host innate responses of induction of inflammasomes and IFN-β.

### BRCA1 is involved in HSV-1 genome recognition by IFI16 during *de novo* infection

Since BRCA1 in complex with IFI16 enhanced the nuclear KSHV genome affinity of IFI16 we further postulated a similar crucial role for BRCA1 in facilitating nuclear HSV-1 genome recognition by IFI16 with concomitant innate response activation. Uninfected HFF cells or HFF cells infected with EdU genome labeled HSV-1 (KOS) with 1 PFU/cell (~25 DNA copies/cell) for 30 min were processed for PLA. Compared to uninfected HFF cells, where BRCA1 was associated with IFI16 only in the nucleus (Fig 13B, green PLA spots) as IFI16 was predominantly present in the nucleus (Fig 13A, green PLA spots), some of the IFI16 and IFI16-BRCA1 PLA spots colocalized with Edu-HSV-1 genome in the nucleus within 30 min of infection (white arrows, Fig 13D and 13E; left and also rightmost panels). Similar to KSHV infection, increased levels of IFI16-BRCA1 spots were observed in the cytoplasm of HSV-1 infected cells (Fig 13E, green spots; yellow arrows). BRCA1 was not associated with ASC in uninfected cells (Fig 13C) and in contrast, BRCA1-ASC association spots were observed in the cytoplasm of HSV-1 infected cells (Fig 13F, green spots; yellow arrows) which suggested that BRCA1 is a constituent of the HSV-1 induced IFI16 inflammasome. More importantly, in BRCA1 knockdown cells, IFI16 was detected only in the nucleus with little colocalization with EdU HSV-1 genome compared to Si-Control cells (Fig 13H vs. Fig 13G).

**Fig 13:** PLA analysis demonstrating the role of BRCA1 in HSV-1 genome recognition by IFI16 during *de novo* infection. Uninfected HFF cells or HFF cells infected with EdU genome labeled HSV-1 (KOS) with 1 PFU/cell (~25 DNA copies/cell) for 30 min were processed for PLA. (**A and D**) PLA reaction (green dots) detecting IFI16 (mouse and goat anti-IFI16 antibodies). (**B and E**) PLA (green dots) detecting the IFI16-BRCA1 complexes. (**C and F**) PLA (green dots) detecting the BRCA1-ASC complexes. The EdU labeled viral genome (red spots) was detected using Alexa 594 labeled azide. Boxed areas in A-C show merged images of nuclei stained with DAPI. The rightmost panels of D-F show merged enlarged images of infected cell nuclei stained with DAPI. White arrows indicate EdU labeled HSV-1 genome (red spots) and its association with IFI16 or IFI16-BRCA1 (PLA green dots). White spots (rightmost panels) represent EdU labeled HSV-1 genome (red spots) and its association with IFI16 or IFI16-BRCA1 (PLA green dots) in the nucleus. Yellow arrows indicate PLA green dots demonstrating IFI16 (D), IFI16-BRCA1 (E) or BRCA1-ASC (F). **(G and H)** Poor association of IFI16 with HSV-1 genomes in BRCA1 knockdown cells. Control Si-RNA (Si-Control) (G) and BRCA1 (Si-BRCA1) (H) knockdown HFF cells were infected with EdU labeled HSV-1 (1 pfu/cell) for 30 min. IFI16 was detected by PLA using mouse and goat anti-IFI16 antibodies. EdU labeled viral genomes were detected by Click-reaction with Alexa 594 labeled azide. Green PLA dots indicate subcellular distribution of IFI16. Yellow arrows: cytoplasmic IFI16. White arrows (yellow spots) indicate association of IFI16 (PLA green dots) with EdU labeled HSV-1 genome (red).

### BRCA1 knockdown results in decreased association of IFI16 with HSV-1 genome during *de novo* infection

To further demonstrate the role of BRCA1 in IFI16 mediated viral genome recognition, we used a biochemical method of DNA mediated chromatin pull down (Fig 14, schematic diagram) [21]. HFF cells pretreated with control Si-RNA or BRCA1 Si-RNA were infected with EdU labeled or unlabeled HSV-1 for 1 h. After protein-DNA cross-linking, biotin-TEG azide was selectively linked to the reactive alkyne group of EdU containing viral DNA via Click reaction. This was followed by DNA shearing, and the small biotin tagged chromatin fragments of HSV-1 genome were captured on streptavidin beads (Fig 14, schematic diagram steps I to V). HSV-1 genome associated IFI16 was analyzed by the elution of streptavidin captured genome bound proteins followed by Western blotting (Fig 14A, schematic diagram step VI). In control Si-RNA treated cells; IFI16 was detected in the eluted fraction from the EdU viral genome pulled down, which suggested the association of IFI16 with HSV-1 genome (Fig 14B, upper 1^st^ panel, lane 3). In contrast, in BRCA1 Si-RNA infected cells, significantly less IFI16 was detected from EdU genome pulled down fractions (Fig 14B, upper 1^st^ panel, lane 4) although similar levels of genome associated histone H3 and TBP were observed in these conditions (Fig 14B, upper 2^nd^ and 3^rd^ panels, lanes 3 and 4). A similar experiment with unlabeled HSV-1 did not detect any protein (Fig 14B, upper panels, lanes1 and 2) pulled down from equal chromatin fractions (Fig 14B, bottom input panels) which demonstrated the specificity of the EdU genome pull down method.

**Fig 14:** Analysis of viral DNA associated host cell proteins by viral DNA mediated chromatin pull down after *de novo* infection with EdU genome labeled HSV-1. **(A)** Schematic diagram representing the strategy for tagging and capturing EdU labeled viral genome and analysis of genome associated proteins. Following preparation of EdU genome labeled HSV-1 (I and II), HFF cells were infected with the labeled virus (10 pfu/cell) for 1 h. After protein-DNA cross-linking (III), biotin-TEG azide was selectively linked to the reactive alkyne group of EdU containing DNA via Click reaction (IV). This was followed by DNA shearing and small chromatin fragments were captured on streptavidin beads (V). These experiments were carried out with unlabeled and labeled virus infection in HFF cells pretreated with control Si-RNA (Si-Control) or BRCA1 Si-RNA (Si-BRCA1). Proteins (VI) and DNA (VII) prepared from these pulled down samples or from input materials were analyzed by western blotting and agarose gel electrophoresis, respectively. **(B)** Detection of viral DNA associated proteins along with inputs by western blotting. **(C)** Agarose gel electrophoresis of the pulled down viral DNA along with input DNA. Arrow: representative pulled down or input DNA is shown.

DNA purified from input and streptavidin captured materials showed similar levels of EdU viral genome pulled down in both control Si-RNA and BRCA1 Si-RNA treated chromatin fractions (Fig 14C, schematic diagram step VII). We also observed that DNA was recovered only from labeled virus infected cells but not from unlabeled virus infected cells (Fig 14C, upper panel, lanes 3 and 4 vs lanes 1 and 2). These studies further demonstrated the specificity of the method.

Overall, these data clearly suggested the involvement of BRCA1 in virus genome recognition by IFI16.

### BRCA1 is necessary for HSV-1 genome recognition induced IFI16-mediated innate inflammasome and type-1 interferon responses during *de novo* infection

We next determined the effect on IFI16 mediated innate immune induction of inflammasomes and IFN-β as a consequence of HSV-1 genome sensing in the presence or absence of BRCA1. Immunoblot analysis from cell lysates of BRCA1 positive (184B5) and BRCA1 negative (HCC1937) cells either uninfected or infected with HSV-1 (1 pfu/cell) demonstrated clear cleavage of caspase-1 and IL-1β at 1, 2 and 4 h p.i. which were nearly absent at 8 h p.i. (Fig 15A, panels 3 and 4, lanes 2–5) which is consistent with IFI16 degradation at later time points p.i. with HSV-1 [5]. In contrast, little or no cleaved caspase-1 or IL-1β was detected in uninfected or HSV-1 infected HCC cell lysates (Fig 15A, panels 4 and 5, lanes 2 and 5 and lanes 7–10). A similar initial increase of pIRF3 at 1, 2 and 4 h p.i. but not at 8 h p.i. was observed in BRCA1 positive HSV-1 infected cells whereas pIRF3 levels were comparatively low or absent in BRCA1 negative cells (Fig 15A, panel 6) with no apparent change in total IRF3 levels (Fig 15A, panel 7). Though HSV-1 infection induced IFI16 at 1 h p.i. (Fig 15A, panel 3), as demonstrated before [5, 7], it was reduced by 2 h p.i. and nearly absent after 4 h p.i. The observed reduction of IFI16, caspase-1, IL-1β and p-IRF3 post HSV-1 infection in BRCA1 positive cells could be due to the increased expression of viral E3 ubiquitin ligase ICP0 (Fig 15A, panel 1) which results in the degradation of IFI16 [5, 7]. In contrast, in the absence of BRCA1, IFI16 levels were not decreased even after 8 h p.i. and actually increased (Fig 15A, panel 3) which could be due to the absence of BRCA1-IFI16 complex resulting in little or no genome recognition by IFI16 and thus unresponsive to ICP0 or some other factors that sequestered IFI16 away from ICP0 leading into delayed degradation kinetics.

**Fig 15:** A crucial role for BRCA1 on host innate immune response activation during HSV-1 infection. BRCA1 (+) and BRCA1 (-) breast tumor epithelial cell lines were infected with HSV-1 at an moi of 1 pfu/cell (**A-D**). (A) Lysates were analyzed by western blots to detect ICP0, BRCA1, IFI16, cleaved caspase-1, cleaved IL-1β, phospho-IRF3 and total IRF3. β-actin was used as a loading control. Supernatants from BRCA1 (+) and BRCA1 (-) cells either uninfected or infected with HSV-1 at an moi of 1 pfu/cell (B and C) for the indicated times were assessed by ELISA for IFN-β (B) and IL-1β (C) release. Results presented are means ± SD (n = 3; * p<0.05, ** p<0.01, *** p<0.001 from BRCA1 (+) vs BRCA1 (-) cells with HSV-1 infection). **(D)** HSV-1 viral yield at 24 h p.i. from BRCA1 (+) and BRCA1 (-) cells originally infected at an moi of 1 pfu/cell (D). (n = 3; * p<0.05 from BRCA1 (-) vs BRCA1 (+) cells with HSV-1 infection). **(E)** Effect of IFI16 knockdown on BRCA1-ASC and ASC-Caspase-1 association during HSV-1 infection. HFF cells treated with control Si-RNA (Si-Control) or IFI16-Si-RNA (Si-IFI16) were infected with HSV-1 (1 pfu/cell) for the indicated times and lysates were IP-ed with anti-ASC antibodies followed by WB with anti-BRCA1 and anti-Caspase-1 antibodies. WCLs were used as input controls for WBs to show IFI16 knockdown, presence of ASC, BRCA1, HSV-1-ICP0 and cleavage of procaspase-1. **(F-G)** Effect of IFI16 knockdown on BRCA1 subcellular distribution. (F) PLA detecting IFI16 in Si-Control or Si-IFI16 treated HFF cells uninfected or infected with HSV-1 (1 pfu/cell) for 2 h. Red dots are indicative of PLA reactions. White arrows: cytoplasmic IFI16. Quantitative analysis of the average number of cytoplasmic IFI16 PLA spots per cell is presented in the rightmost columns. ***: p<0.001. (G) PLA detecting BRCA1 in a similar condition as F. Green dots indicate PLA reactions representing subcellular distribution of BRCA1. White arrows: cytoplasmic BRCA1. Quantitative analysis of the average number of cytoplasmic BRCA1 PLA spots per cell is presented in the rightmost columns. ***: p<0.001.

HSV-1 infection in BRCA1 positive cells resulted in an initial increase in secreted IFN-β and IL-1β at 2 h and 4 h p.i. followed by a decrease at 8 h p.i. (Fig 15B and 15C) which were significantly reduced in BRCA1 negative cells (Fig 15B and 15C). Interestingly, similar to our earlier observation in IFI16 negative cells [9], compared to BRCA1 positive cells, >4 fold increase in HSV-1 yield was observed in BRCA1 negative cells upon HSV-1 infection (Fig 15D). This could be either due to less IFN-β production as a result of the absence of an IFI16-STING-TBK1-IRF3 signal cascade or loss of inflammasome activation in these cells and/or decreased transcriptional repressor activity of IFI16 as a result of decreased viral genome affinity of IFI16.

Furthermore, in the co-IP experiments, BRCA1 and Caspase-1 were detected in ASC immunoprecipitates from Si-Control RNA treated HSV-1 infected (1 pfu/cell) HFF cells. In contrast, little or no BRCA1 or Caspase-1 were co-IP-ed with ASC in IFI16 knockdown (Si-IFI16) cells (Fig 15E, 1^st^ and 2^nd^ panels) and the presence of cleaved Caspase-1 was observed only in control-Si-RNA treated HSV-1 infected cells (Fig 15E, 5^th^ panel). Whole cell lysates from Si-Control and Si-IFI16 HFF cells (Fig 15E, 3^rd^ panel) showed BRCA1, ASC, Caspase-1 and HSV-1-ICP0 levels (Fig 15E, panels 4, 5, 6 and 8).

When we analyzed the BRCA1 cellular distribution in IFI16 knockdown HFF cells infected with HSV-1 for 2 h (Fig 15F and 15G), as observed before, IFI16 PLA spots were detected in the nucleus and in the cytoplasm of infected cells which were significantly absent in the Si-IFI16 cells which demonstrated the efficiency of IFI16 knockdown (Fig 15F). Compared to uninfected Si-control cells with some amount of BRCA1 in the cytoplasm, HSV-1 infection resulted in significantly increased BRCA1 cytoplasmic distribution which was significantly reduced in the IFI16 knockdown virus infected cells with a level comparable to that of the uninfected cells (Fig 15G and bar graph).

These results suggested the dependence on IFI16 for the observed BRCA1-ASC and ASC-Caspase-1 association during inflammasome complex formation and increased cytoplasmic BRCA1 translocation during HSV-1 infection. These results also clearly demonstrated that similar to KSHV, BRCA1 is also essential for IFI16 to sense the HSV-1 genome, activation of inflammasomes, cytoplasmic translocation, and in the induction of the IFN-β response.

## Discussion

The innate immune system of mammalian cells utilizes distinct sensors and methods to detect DNA in endosomes, cytoplasm, or the nucleus which include recognizing differences in physicochemical structure such as CpG motifs or AT-rich regions of microbial DNA, abnormal occurrence of microbial DNAs or accumulation of endogenous or microbial DNA and elicitation of DDR against incoming viral DNAs [22]. Our studies presented here reveal that formation of distinct complexes, such as IFI16-BRCA1, is another way to detect herpes viral DNA entering the nucleus. These comprehensive studies demonstrate that BRCA1 plays a hitherto unidentified role as a cofactor to IFI16 in the nuclear innate sensing of foreign DNA and subsequent assembly and cytoplasmic distribution of stable IFI16-inflammasomes leading into IL-1β formation as well as the induction of IFN-β via cytoplasmic signaling through IFI16, STING, TBK1 and IRF3 (Fig 16).

**Fig 16:** Schematic model depicting the proposed role of BRCA1 in the IFI16-mediated viral DNA genome sensing and innate immune response activation during KSHV, HSV-1 and EBV infection of target cells. (**1**) Following viral entry, the nucleocapsid traffics to the nuclear pore region, linear DNA enters into the nucleus and circularizes to form episomal DNA. (**2**) Sequence-independent sensing of viral DNA by the DNA binding HIN-domain of IFI16 likely requires a pre-existing complex with BRCA1. BRCA1 forms this complex via association with the PYD domain of IFI16, which predisposes IFI16 as a dedicated viral DNA sensor, leading to the IFI16 mediated innate immune activation, one arm of which results in inflammasome activation (**2–7**) and the other arm initiates cytoplasmic immune signaling resulting in IFN-β/type I IFN induction (**i-vii**). Viral genome sensing by the BRCA-IFI16 complex recruits the adaptor protein ASC and procaspase-1 for the assembly of an inflammasome complex (**3**). This is followed by inflammasome translocation to the cytoplasm (**4**), to produce functionally active Caspase-1 (**5**), and subsequent cleavage of pro-IL-1β into mature IL-1β (**6**) for secretion (**7**). Increased BRCA1-IFI16 association during early as well as late times of *de novo* KSHV,EBV and HSV-1 infection and during latent KSHV and EBV infection, subsequent inflammasome activation and reduced IFI16-ASC-Caspase-1 inflammasome assembly in the absence of BRCA1 demonstrate a continuous sensing of viral genome by the BRCA1-IFI16 complex and thus provides a hitherto unidentified role of BRCA1 as a critical cofactor in the initiation of the IFI16-inflammasome. The IFI16-BRCA1 complex not involved in inflammasomes also translocates to the cytoplasm during *de novo* KSHV and HSV-1 infection (**i**) and interacts with STING to induce innate immune signaling (**ii**) via the IFI16-STING-TBK1 axis resulting in IRF3 phosphorylation (**iii**) and subsequent nuclear translocation (**iv**) leading to IFN-β transcription (**v**), IFN-β production (**vi**) and secretion (**vii**).

Similar to the IFI16-BRCA1 interaction, previous studies suggest that some of the cytoplasmic inflammasome sensor molecules require cofactors to recognize their ligands or to be stabilized in their activated states. For example, NLRP1 requires NOD2 protein to interact with muramyl dipeptide ligand and to activate the NLRP1 inflammasome [23]. NLRC4 inflammasome formation requires NAIP (NLR family, apoptosis inhibitory protein). Mouse NAIP5 and NAIP6 detect flagellin, NAIP2 senses the type III secretion component Prg J and human orthologue NAIP senses a type III secretion needle protein to activate the NLRC4 inflammasome [24]. Similarly, formation of the NLRP3 inflammasomes in response to non-crystalline activators is also promoted by guanylate-binding protein 5 [25].

The presence of foreign microbial or host DNA in the cytoplasm is recognized as abnormal by AIM2 resulting in the AIM2-inflammasome [26]. Studies of the crystal structures of HIN domains of AIM2 and IFI16 in complex with dsDNA demonstrated that IFI16 and AIM2 recognize DNA in a non-sequence specific manner through electrostatic attraction between the positively charged HIN domain residues and the sugar phosphate backbone of dsDNA. In these studies with overexpressed proteins out of context of the nuclear environment, the PYD and HIN domains of AIM2 are shown to be in an autoinhibited intramolecular complex state which is liberated upon DNA binding thus facilitating DNA-mediated assembly of an inflammasome along the DNA staircase [1]. Whether AIM2 requires additional factor(s) for its function in the cytoplasm is not known.

In the nucleus, the nuances of sequence independent DNA sensing by IFI16 distinguishing between foreign and host DNA are not clear, since unlike other danger signals inducing inflammasomes and the interferon response, DNA is not unique to pathogens. Our studies demonstrate that the BRCA1 interaction with IFI16 predisposes IFI16 to recognition of viral genome as shown by the less IFI16 association in viral EdU genome pull down analysis and poor colocalization of IFI16 with EdU viral genome in the BRCA1 knockdown cells. Hence, the interaction of BRCA1 with the pyrin domain of IFI16 [15,19] could be liberating the autoinhibited complex state thus facilitating the HIN domains of IFI16 to sense the viral genome to trigger a rapid inflammasome and interferon-β response.

A recent study suggested that the PYD domain is essential for driving IFI16 to cooperatively assemble into filaments on DNA when IFI16 encounters long dsDNAs (greater than 20 bp in size), which can elevate the dsDNA binding efficiency of IFI16 [27]. In the nucleus, the major exposed self-dsDNAs are thought to be the dsDNA linkers between nucleosomes or the transcription bubbles, which are about 20 bp in size [28, 29]. It is believed that the exposed self-dsDNA in such short lengths would bind nuclear IFI16 with limited affinity and would not be capable of providing a sufficient platform for IFI16 to oligomerize into filaments or inflammasomes, thereby preventing spurious activation of immune pathways [27]. In contrast, IFI16, already in an open conformation aided by the interaction of BRCA1 with the PYD domain, probably rapidly engages the non-chromatinized dsDNA viral genomes of KSHV, EBV and HSV-1 soon after their nuclear entry more efficiently than self-DNAs likely due to a higher binding affinity leading to the rapid assembly of IFI16 inflammasomes and induction of the IFN-β response. Non-availability of BRCA1 may render a limited IFI16 response/affinity for such exposed viral DNA, which is insufficient to induce inflammasome activation and IFN-β production.

The immunomodulatory role of IFI16 is shown by its ability to recognize and respond to the presence of nuclear herpesviral and non-integrated HIV genomes, leading to inflammasome induction and/or to participate in STING-mediated IFN-β expression during HSV-1 and vaccinia virus infection [30]. Although IFI16 was demonstrated to interact with cytoplasmic STING in a DNA-dependent manner resulting in the recruitment of TBK1 and IRF3 plus phosphorylation of IRF3 [1,6], the key unresolved question concerns the mechanisms by which nuclear DNA sensing by nuclear resident IFI16 can trigger cytosolic STING dependent IFN-β induction. This would either require delivery of IFI16 as a nuclear IFI16-DNA complex to the cytoplasm for direct association with STING or for a cGAS (cGAMP-Synthase)-mediated cGAMP (cyclic GMP-AMP) production to bind with STING [31]. Absence of viral genome in the cytoplasm of productively infected cells together with the near absence of IFI16-STING in the BRCA1 knockdown cells infected with KSHV or HSV-1 clearly suggest the formation of a distinct IFI16 molecular complex with one or more nuclear protein(s), such as BRCA1, drives IFI16’s cytoplasmic trafficking, leading to the interaction of IFI16 with the STING signalosome.

Although initially identified as a cytoplasmic DNA sensor [31], in a recent study, Orzalli *et al*., [32] reported the detection of cGAS in both the nucleus and cytoplasm of HFF and immortalized oral keratinocyte cells. IFI16 was detected in HEK293 cells and not in 293T cells, and cGAS was absent in HEK293 and 293T cells. Knockdown of both cGAS and IFI16 reduced the IFN-β responses in HSV-1 infected HFF cells. IFI16 appeared to be stabilized by cGAS in the uninfected HFF cells as in the absence of cGAS, IFI16 half-life was moderately reduced [32]. The endogenous IFI16 co-precipitated with cGAS from the whole cell extracts of normal as well as HSV-1 infected HFF cells (3 h p.i.). However, whether this interaction occurs in the nucleus or in the cytoplasm and the kinetics of this interaction after nuclear viral genome recognition is not known. From the observations of the localization of IFI16 at the site of Wt-HSV-1 (KOS) viral genome and replication and the absence of cGAS at this site, Orzalli *et al*., [32] have concluded that IFI16 is the primary sensor of viral DNA in the nucleus and cGAS is not involved in genome recognition. They also reported that cGAS is involved in the early induction of the IFN-β response against transfected DNA, probably by recognizing the DNA in the cytoplasm and is also required for the IFN-β response at 8 h post-HSV-1 infection. Inflammasome response against the transfected DNA by AIM2 was not examined. In addition, how the message of nuclear viral genome sensing by IFI16 in the presence of nuclear cGAS is transmitted to the cytoplasm for STING-IRF3 mediated IFN-β production is not clear. Our studies suggest that IFI16 requires BRCA1 to increase its affinity to nuclear viral DNA leading into the sustained innate responses including the translocation of IFI16 into the cytoplasm of infected cells and the activation of STING. Unlike cGAS, which has transient association with IFI16 [32], our studies show that BRCA1 is associated with IFI16 in the nucleus under physiological conditions, and is involved in the sensing of herpes viral (KSHV, EBV and HSV-1) genomes by IFI16 and in the consequent innate inflammasome and IFN-β responses. It is likely that the interaction of IFI16 and STING is within a complex in the cytoplasm that may be stabilized by cGAS. Whether cGAS interacts with IFI16-BRCA1 or not and the kinetics, as well as the role of cGAS in IFI16-BRCA1-STING mediated innate IFN-β response requires additional studies which are beyond the scope of the present study.

A recent study utilized a PMA stimulated human monocytic THP-1 cell line for infection with KSHV and reported that IL-1β and IFN-β were induced via an IFI16 independent pathway [30]. However, the authors did not demonstrate that the TPA stimulated THP-1 cell actually supported KSHV and HSV-1 infection, and both viruses are known to infect unstimulated THP-1 cells. Moreover, due to increased phagocytosis in PMA induced THP-1 cells, herpesviruses undergo abortive infection, resulting in the accumulation of virus particles in lysosomes and the release of viral DNA to the cytoplasm [33]. This DNA is likely recognized by AIM2 and cGAS, to stimulate the IL-1β and interferon responses. In contrast, during *in vitro* infection of permissive cells, viral DNA from the capsid enters the IFI16 rich nucleus resulting in the consequences presented by our studies.

Besides the role of IFI16 in inflammasome and type 1 IFN induction, IFI16 is also shown to be a transcriptional modulator; however, the detailed mechanisms are poorly defined [16]. Recent studies by us and others demonstrated that in HSV-1 infected cells, IFI16 promoted the addition of repressive heterochromatin H3K9me3 markers and reduced the active euchromatin H3K4me3 markers on the viral gene promoters resulting in the reduced binding of transcription factors Oct1 and TBP, plus RNA pol II [8, 9]. Studies suggest that IFI16 may target exogenous DNA not associated with nucleosomes as virion associated dsDNA of SV40 genome containing nucleosomes and the adenoviral genome with core protein VII were resistant to the restriction effect of IFI16 [7]. However, from our studies showing that IFI16 is associated with latent chromatinized KSHV and EBV genomes, continuation of viral latent gene expression in the presence of IFI16 and IFI16-inflammasomes [3, 4], IFI16’s ability to mediate global differences in HSV-1 genome chromatin modifications [8, 9], and our ongoing studies showing the binding of IFI16 to the KSHV gene promoters in latently infected cells, we theorize that IFI16 has very complex roles in gene regulation and there may be other factors involved in IFI16’s ability to discriminate foreign vs. host DNA. Similar to the IFI16-BRCA1 complex involved in pathogen DNA recognition, inflammasome induction and IFN-β production shown here, it is possible that IFI16 could be forming distinct complexes with different proteins and each complex could be mediating distinct functions, such as transcription and other responses, which may differ between various virus nuclear lytic and latent infections and as per host cell types. Determining these possibilities and deciphering whether BRCA1 plays a role in IFI16’s ability to influence viral promoters and in the nuclear life cycles of DNA viruses requires further extensive studies which are beyond the scope of the present study.

Lack of association of BRCA1 with ASC in IFI16 knockdown cells demonstrated that BRCA1 likely doesn’t interact directly with ASC but relies on IFI16 for ASC association and for subsequent stable inflammasome formation. The multiple binding sites of ASC-PYD with distinct positively and negatively charged surfaces are proposed to transition between folded and unfolded states to regulate PYD function [34, 35]. The interaction of BRCA1 with the PYD of IFI16 could facilitate the spatial distribution of the binding sites between IFI16 and ASC to drive their stable association and inflammasome assembly. BRCA1 knockdown significantly reduced cytoplasmic IFI16 suggesting that BRCA1 facilitates cytoplasmic trafficking of nuclear IFI16 during KSHV and HSV-1 infection, which could be due to BRCA1 dependent post-translational modification (acetylation or phosphorylation) of IFI16. Different IFI16 motifs have been demonstrated to regulate IFI16 subcellular localization [36], and the role of BRCA1 in post-translational modification and cytoplasmic distribution of IFI16 are under investigation.

BRCA1 has been reported to be distributed in the nucleus and cytoplasm with distinct functionality such as DDR, chromatin remodeling, checkpoint control and apoptosis [37]. However, less cytoplasmic BRCA1 in IFI16 knockdown than control Si-RNA treated virus infected cells observed by us probably demonstrates the need for IFI16 in complex with BRCA1 for viral genome sensing followed by translocation to the cytoplasm. Although a study suggests the role of BRCA1-IFI16 interaction in a p53-mediated apoptosis pathway [15], IFI16 or BRCA1 knockdown did not affect endothelial cell viability. As shown here, formation of the IFI16-inflammasome was not detected in cells induced for DDR by bleomycin. Furthermore, the presence of DDR proteins CHK2 and H2AX in BRCA1 immunoprecipitates, but not in IFI16 immunoprecipitates despite the increased BRCA1-IFI16 interaction during KSHV infection, suggests that the BRCA1-IFI16 complex is probably not related to host DDR or apoptosis responses during DNA virus infection and may have evolved to mediate innate sensing and other functions.

The protective immune response triggered by the detection of microbial effectors termed “effector triggered immunity (ETI)” enables the host to distinguish pathogens from non-pathogen [38, 39, 40] and this is probably of relevance in non-professional immune cells too, such as epithelial, endothelial and other cells that come in contact with pathogens at different *in vivo* sites, including at the portal of pathogen entry. Our studies demonstrating that IFI16-BRCA1 functions as an innate sensor of KSHV, EBV and HSV-1 genomes in non-immune professional cells, such as endothelial, epithelial and fibroblast cells, and in B-lymphoma cell lines as well as the IFI16 and ASC interactions in tissue sections from PEL and KS patients [3], clearly suggested that these cells have evolved to respond to danger signals. Additional studies are required for a clear understanding of the molecular mechanism of BRCA1 and IFI16 in the fundamental relation between innate DNA sensing, viral and host genome regulation, chromatin remodeling, inflammation and immunity.

## Materials and Methods

### Cells

HMVEC-d and HFF cells (Clonetics, Walkersville, MD), TIVE, TIVE-LTC, BCBL-1, LCL, BJAB, Akata, Ramos, and BRCA1 positive and negative breast carcinoma (ATCC CRL 8799 and 2336) cells were grown as described before [2,4,41].

### Viruses

#### KSHV

Induction of the lytic cycle in BCBL-1 cells by phorbol ester, supernatant collection, and virus purification were described previously [2]. KSHV DNA was extracted, copy numbers quantitated by real-time DNA-PCR, and infection was done with 30 genome copies/cell [2].

#### HSV-1

HSV-1 (KOS) propagation and viral titer by plaque assay on Vero cells were done as described [5]. Briefly, Vero cells were infected with HSV-1 (0.001 pfu/cell), collected at 3–5 days, cells removed by centrifugation at 1,000 rpm for 10 min at 4°C, supernatant virus pelleted by centrifugation at 20,000xg for 2 h at 4°C, pellet resuspended in PBS-AB/15% glycerol and stored at -80°C.

#### EBV

The EBV lytic cycle in LCL cells was induced with *n*-butyric acid at a final concentration of 3 mM for 4 days. Cells were centrifuged at 1,800 × *g* for 20 min, and the supernatant was filtered through a 0.45-mm-pore-size cellulose acetate filter. EBV viral particles were concentrated by ultracentrifugation at 70,000 ×*g* at 4°C, and virus pellets were suspended in RPMI medium without serum in 1/100 volume of original medium [4].

### BrdU or EdU genome labeled virus

KSHV DNA was metabolically labeled during lytic replication by adding the thymidine analogue 5-Bromo-2’-deoxyuridine (BrdU) (Life Technologies) (1:100 v/v from supplied stock) or 5-ethynyl-2’-deoxyuridine (EdU) (Sigma) (10 μM) in DMSO to the culture medium of BCBL-1 cells on day 1 and day 3 of phorbol ester induction, and labeled virus from the day 5 culture supernatant was purified and genome copy numbers determined [2]. HSV-1 (KOS) genome was labeled by adding EdU to the Vero cell medium at 8 h, day 1 and 2 post-infection and labeled virus in the day 4 supernatant was purified and titer determined [5].

### Virus infection

#### KSHV

Cells were incubated with 30 KSHV DNA genome copies/cell for 2 h or the time indicated, washed to remove uninternalized virus and incubated for different time periods [2].

#### Vaccinia

HMVEC-d cells were infected with vaccinia virus at an moi of 5 pfu/cell for 2 h, washed and incubated with complete media for 8 h until processed for the experiment [2].

#### HSV-1

Cells were incubated with HSV-1 (1 pfu/cell; ~25 DNA genome copies/cell) in serum free medium for 2 h or until the time indicated, washed and incubated in DMEM supplemented with 2% FBS for the indicated time periods, and viral yield at 24 h p.i. was determined by plaque assay [9].

### Primary KSHV and EBV infection of human PBMCs

Deidentified peripheral blood mononuclear cells (PBMCs) were obtained from the University of Pennsylvania CFAR Immunology Core, and 1 × 10^7^ PBMCs were infected [4]. Briefly, PBMCs were infected with KSHV or EBV in 1 ml of RPMI 1640 medium with 10% FBS and 5 ng/ml of Polybrene (Sigma, Marlborough, MA). After 4 h at 37°C (time point 0), infected and uninfected cells were centrifuged for 5 min at 1,200 × *g*; the pellet was washed twice with fresh RPMI medium, resuspended in fresh RPMI medium with 10% FBS, and cultured in six-well plates at 37°C. These cells were collected at different times p.i., and washed twice with 1× phosphate-buffered saline (PBS) before being spotted on slides.

### Antibodies (Table 1)

Mouse monoclonal antibodies against human BRCA1 and rabbit polyclonal antibodies against human BRCA1 were from GeneTex, Irvine, CA and Millipore, Billerica, MA, respectively. Rabbit anti-human H2AX, γH2AX and CHK2 antibodies were from Cell Signaling Technology, Beverly, MA. Mouse monoclonal antibodies against human ASC were from MBL International, Woburn, MA. Goat polyclonal antibodies against human ASC/TMS1 were from Ray Biotech, Norcross, GA. Mouse monoclonal anti-IL-1β antibodies were from R&D Systems, Inc., Minneapolis, MN. Rabbit, mouse and goat antibodies against human IFI16 were from Sigma, St Louis, MO and Santa Cruz Biotechnology, Inc., respectively. Rabbit polyclonal anti-caspase-1 antibodies were from Bio Vision, Milpitas, CA. Rabbit anti-AIM2 and mouse anti-NLRP3 antibodies were from Abcam Inc., Cambridge, MA. Rabbit monoclonal antibodies against STING, p-IRF3 and Histone H3 are from Cell Signaling Technology. Mouse monoclonal anti-IRF3 antibody was from Abcam Inc. Alexa 594 or 488 anti-rabbit and anti-mouse secondary antibodies were from Molecular Probes, Invitrogen, Carlsbad, CA. Anti-rabbit and anti-mouse antibodies linked to horse-radish peroxidase were from KPL Inc., Gaithersburg, MD. Mouse monoclonal antibodies against β-actin and β-tubulin were from Sigma. Mouse monoclonal anti-TATA binding protein (TBP) antibody was from Abcam Inc. Protein A-Sepharose 6 MB and Protein G-Sepharose CL-4B Fast Flow beads were from Amersham Pharmacia Biotech, Piscataway, NJ.

### Nuclear and cytoplasmic extract preparation

Cells were harvested and used for preparation of nuclear and cytoplasmic extracts using a nuclear extract kit (Active Motif Corp., Carlsbad, CA) as per the manufacturer's instructions. After measurement of protein concentrations with BCA protein assay reagent (Pierce, Rockford, IL), nuclear and cytoplasmic extracts were subjected to Western blot (WB) analysis with different antibodies. The purity of the nuclear extracts and cytoplasmic extracts was assessed by immunoblotting with anti-TBP and anti-β-tubulin antibodies, respectively.

### Western blot analysis

Cells were lysed in radioimmunoprecipitation assay (RIPA) lysis buffer (15 mM NaCl, 1 mM MgCl2, 1 mM MnCl2, 2 mM phenylmethylsulfonyl fluoride and protease inhibitor mixture (Sigma)), sonicated, and centrifuged at 10,000 rpm at 4°C for 10 min. Protein concentrations were estimated by BCA protein assay reagent (Pierce). Equal concentrations of proteins were separated by SDS-PAGE, transferred to nitrocellulose and probed with the indicated specific primary antibodies followed by incubation with species-specific HRP-conjugated secondary antibody and chemiluminiscence based detection (Pierce) of immunoreactive protein bands according to the manufacturer’s protocol. Blots were scanned and quantitated using FluorChemFC2 software and an AlphaImager system (Alpha Innotech Corporation, San Leonardo, CA).

### Immunoprecipitation

Cells were lysed in lysis buffer (25 mM Tris-HCl, pH: 7.5, 150 mM NaCl, 1% NP40, 2 mM EDTA, 10% Glycerol, and protease inhibitor mixture). Two hundred μg of clarified and precleared cell lysate proteins were incubated overnight with immunoprecipitating antibody at 4°C, the resulting immune complexes were captured by protein A- or G-sepharose and analyzed by western blotting, using specific detection antibodies.

### RNA interference using Si-RNA transfection

Transfection of primary HMVEC-d and HFF cells with siRNA was performed using a Neon Transfection System (Invitrogen) according to the manufacturer’s instructions. Briefly, subconfluent cells were harvested and washed once with 1x phosphate-buffered saline (PBS) and resuspended at a density of 1 x10^7^ cells/ml in resuspension buffer R (provided by the company). Ten microliters of this cell suspension was mixed with 100 pmol of Si-RNA and then microporated at room temperature using a single pulse of 1,350 V for 30 ms for HMVEC-d and 1,700 V for 20 ms for HFF. After microporation, cells were distributed into complete medium and placed at 37°C in a humidified 5% CO2 atmosphere. At 48 h post-transfection, cells were analyzed for knockdown efficiency by Western blotting. All Si-RNA oligonucleotides (siGenome SMARTpool) for BRCA1, IFI16 and non-targeting Si-RNA pool no. 2 were purchased from Thermo Scientific (catalog no. M-003461-02-0010, M-020004-01-0010, and D-001206-14-20).

### Immunofluorescence microscopy

HMVEC-d cells were seeded on glass 8-well chamber slides (Nalgene Nunc International, Naperville, IL) and uninfected or KSHV infected (30 DNA copies/cell or latently infected) cells were fixed for 15 min with 4% paraformaldehyde, and permeabilized with 0.2% Triton X-100 for 5 min. Cells were then washed and blocked with Image-iT FX signal enhancer (Life Technologies) for 20 min. The cells were reacted with primary antibodies against the specific proteins, followed by fluorescent dye-conjugated secondary antibodies. To detect EdU labeled viral genome, cells were fixed, permeabilized and blocked with Image-iT FX signal enhancer (Life Technologies) for 20 min. A CLICK reaction was performed for 30 min at RT using Click-iT EdU reaction additive (Life Technologies), EdU reaction buffer, copper sulphate and Alexa Fluor 594 azide. Cells were observed by Nikon Eclipse 80i microscope, and analyzed with Metamorph digital imaging software. All experiments were performed three independent times and three different fields with a minimum of 20 cells were analyzed. All images were acquired at 40 X magnification.

### BRCA1 lentiviral expression in BRCA1-null HCC1937 cells

BRCA1 (Human) Gateway V5-tagged lentiviral expression vector (pLX304) was from DNASU Plasmid Repository (Arizona State University Biodesign Institute, Tempe, AZ). BRCA1 lentivirus was produced using a four plasmid transfection system as previously described [42]. Briefly, 293T cells were transfected with BRCA1 expressing vector and packaging plasmids and the media was changed 16 h after transfection. Supernatants containing packaged lentivirus were collected at 48 h, passed through a 0.45 μm filter and used to transduce BRCA1 negative cells (HCC 1937) in the presence of polybrene (5 μg/ml, Pierce, Rockford, IL). 48 h post-transduction with control lenti and BRCA1 lenti expression vectors, cell lysates were processed for IP and Western blotting.

### IL-1β ELISA

Secretion of IL-1β was detected using Ray Bio Human IL-1β ELISA Kit (Ray Biotech, Norcross, GA) according to the manufacturer’s instructions. Supernatant from uninfected or virus infected cells (~3X10^5^) was collected at different times p.i., incubated in the assay wells overnight at 4°C, washed, incubated 1 h with the biotinylated antibody, and with HRP conjugated streptavidine solution at room temperature for 45 min. Wells were washed, incubated with TMB substrate in the dark for 30 min at room temperature followed by addition of stop solution, and the absorbance at 450 nm was read using a Synergy2 Biotek Plate Reader (Biotek, Winooski, VT).

### IFN-β ELISA

IFN-β secretion levels were measured using the *Verikine* Human IFN Beta ELISA kit (PBL, Interferon Source, Piskataway, NJ) according to the manufacturer’s instructions. Supernatants from uninfected or virus infected cells (~3X10^5^) were collected at different times post-infection, diluted 1:1 with sample dilution buffer and incubated in the assay wells at room temperature for 1 h [9].

### Proximity ligation assay microscopy

A DUOLink PLA kit (Sigma) was used to detect protein–protein interactions. HMVEC-d and HFF cells were cultured and infected with KSHV (30 DNA copies/cell) in 8 chamber microscope slides, fixed in 4% PFA for 15 min at room temperature, permeabilized with 0.2% Triton X-100 and blocked with Duolink blocking buffer for 30 min at 37°C. TIVE and TIVE-LTC cells were fixed, permeabilized and blocked with Duolink blocking buffer as described above. Equal numbers of BJAB, BCBL-1, Akata, Ramos and LCL cells were washed extensively with PBS by centrifugation at 200xg at 4°C and spotted on 10-well glass slides and were fixed/permeabilized with prechilled acetone and blocked with Duolink blocking buffer. Cells were incubated with primary antibodies diluted in Duolink antibody diluents for 1 h, washed and then further incubated for another 1 hr at 37°C with species specific PLA probes (PLUS and MINUS probes) under hybridization conditions and in the presence of 2 additional oligonucleotides to facilitate hybridization of PLA probes only if they were in close proximity (<40 nm). A ligation mixture and ligase were then added to join the two hybridized oligonucleotides to form a closed circle. Several cycles of rolling-circle amplification using the ligated circle as a template were performed by adding an amplification solution to generate a concatemeric product extending from the oligonucleotide arm of the PLA probe. Lastly, a detection solution consisting of fluorescently labeled oligonucleotides was added, and the labeled oligonucleotides were hybridized to the concatemeric products. The signal was detected as a distinct fluorescent dot in the Texas red or FITC green channel and analyzed by fluorescence microscopy. Specificity of PLA was determined by using negative controls consisting of samples treated as described but with only secondary antibodies. An additional series of negative control PLA was conducted using each single species primary antibody followed by incubation with both species secondary antibodies. PLA was quantified using DUOLink software.

For *in situ* double sequential PLA of IFI16-BRCA1 and IFI16-ASC complexes, two independent PLA reactions were performed sequentially. Briefly, the PLA reaction for IFI16 and BRCA1 was performed first using rabbit anti-IFI16 and mouse anti-BRCA1 antibodies and detected by DUOLink red detection agent. Cells were then washed, blocked with PLA blocking buffer and subjected to a second PLA reaction using mouse anti-IFI16 and goat anti-ASC antibodies and detected with DUOLink green detection agent.

### EdU labeled HSV-1 viral DNA mediated chromatin pull down assay

For EdU-labeled genome (chromatin) pull down, we used methods described by Kliszczak *et al*. [21] with minor modifications. Briefly, HFF cells (8 X 10^6^) pretreated with control Si-RNA or BRCA1 Si-RNA for 72 h were infected with unlabeled or EdU labeled HSV-1 (10 pfu/cell) for 1 h and then cross-linked with 1% formaldehyde for 10 minutes at 4°C. Unreacted formaldehyde was quenched with the addition of 0.125 M glycine for 10 minutes at 4°C. Cells were harvested and permeabilized with 0.1% (v/v) Triton X-100 in PBS for 10 minutes on ice and washed with PBS. Biotin was attached to EdU genome via Click reaction with sequential addition of the following reagents, 10 mM (+)-sodium-L-ascorbate, 0.1 mM biotin-TEG azide and 2 mM copper (II) sulfate followed by 30 minutes incubation in the dark at room temperature and by addition of 10 volumes of 1% (w/v) BSA, 0.5% (v/v) Tween 20 in PBS for 10 minutes. After three PBS washes, soluble proteins were extracted in 500 μl CL lysis buffer (50 mM HEPES, pH 7.8, 150 mM NaCl, 0.5% (v/v) NP-40, 0.25% (v/v) Triton X-100, 10% (v/v) glycerol) with protease inhibitors by end-over-end mixing at 4°C for 10 minutes and then slow speed centrifugation (1800 rpm / 300 x g). The pellet was washed with 500 μl wash buffer (10 mM Tris-HCL pH 8.0, 200 mM NaCl, 0.5 mM DTT) for 10 minutes at 4°C by end-over-end mixing. Following low speed centrifugation, the pellet was then resuspended in 500 μl RIPA buffer (10 mM Tris-HCl, pH 8.0, 140 mM NaCl, 1% (v/v) Triton X-100, 0.1% (v/v) Na-Deoxycholate, 0.1% (w/v) SDS) with protease inhibitor cocktail and processed for shearing of the chromatin via sonication on ice at an amplitude of 40, 10 seconds on, 10 seconds off for 10 minutes. The extract was clarified by centrifugation at 15,000 x g for 10 minutes at 4°C. Protein content was quantitated and 30 μg of the supernatants were used for input western blotting. 1 mg of the extract was used for pull down with 50 μl of streptavidin magnetic beads which were washed with wash buffer, equilibrated with RIPA buffer and blocked overnight at 4°C with 0.5 mg/ml BSA and 0.4 mg/ml presheared salmon sperm DNA to minimize non-specific binding. Next day, beads were washed with wash buffer and incubated with chromatin extracts for 8 h at 4°C. Beads with bound complexes were then washed with wash buffer and subjected to reverse protein-DNA cross-linking and elution of proteins by incubation with 1X *Laemmli* sample buffer for 10 minutes at 95°C before SDS-PAGE. For DNA purification, complexes from beads were eluted in elution buffer (1% SDS; 0.1M NaHCO3). The cross-linking was reversed by treatment with 0.1 mg/ml RNase A and 0.3 M NaCl at 37°C for 30 minutes followed by incubation at 65°C for 2 h with 0.1 mg/ml Protenase K and DNA was column purified via Qiagen DNA extraction kit according to manufacturer’s instructions.

### Statistical analysis

Data are expressed with means ± SD of at least three independent experiments (n≥3) using a Student’s T-test. In all tests, *p*<0.05 was considered statistically significant. Experiments in which p is <0.05 are marked with a single asterisk and *p*<0.01 are marked with double and *p*<0.001 with triple asterisks.

## Supporting Information

S1 Fig Specificity controls for PLA in untreated or bleomycin treated HMVEC-d cells. Cells were washed, fixed, permeabilized and reacted first with either anti-IFI16, BRCA1, CHK2, γH2AX or ASC antibodies alone (indicated as PLA control IFI16; PLA control BRCA1; PLA control γH2AX; PLA control ASC and PLA control CHK2, respectively) and then with 2 secondary antibodies linked to PLA probes (positive probe and negative probe) for the PLA reaction. Nuclei were stained with DAPI. Inset shows enlarged image of a representative cell.
(TIF)

S2 Fig Specificity controls for proximity ligation assay to detect interactions between IFI16, BRCA1, ASC and Caspase-1 in KSHV infected HMVEC-d cells. **(A-E)** HMVEC-d cells were infected with KSHV (30 DNA copies/cell) for 2 h, washed and further incubated for 24 h. Cells were washed, fixed, permeabilized and reacted first with either anti-IFI16, BRCA1, Caspase-1 or ASC antibodies alone and then with two secondary antibodies linked to PLA probes (positive probe and negative probe) as follows; (A) 1^0^ ab: mouse anti-IFI16, 2^0^ abs: anti-mouse probe + and anti-rabbit probe; (B) 1^0^ ab: rabbit anti-IFI16, 2^0^ abs: anti-mouse probe + and anti-rabbit probe; (C) 1^0^ ab: mouse anti-BRCA1, 2^0^ abs: anti-mouse probe + and anti-rabbit probe; (D) 1^0^ ab: Rabbit anti-Caspase-1, 2^0^ abs: anti-mouse probe + and anti-rabbit probe; (E) 1^0^ ab: Goat anti-ASC, 2^0^ abs: anti-mouse probe + and anti-goat probe. PLA reaction was detected using DUOLink Red detection reagent. The absence of any red spots indicates the absence of any PLA reaction when any primary antibody was used alone, suggesting specificity of the PLA signals observed as shown in main Fig 2C–2G. Nuclei were stained with DAPI.
(TIF)

S3 Fig Effect of IFI16 knockdown on BRCA1 subcellular distribution during KSHV infection. **(A)** PLA detecting IFI16 in Si-Control or Si-IFI16 treated HMVEC-d cells uninfected or infected with KSHV (30 DNA copies/cell) for 4 h. Red dots are indicative of PLA reactions. White arrows: cytoplasmic IFI16. Quantitative analysis of the average number of cytoplasmic IFI16 PLA spots per cell is presented in the rightmost columns. ***: p<0.001. **(B)** PLA detecting BRCA1 in a similar condition as in A. Green dots indicate PLA reactions representing subcellular distribution of BRCA1. White arrows: cytoplasmic BRCA1. Quantitative analysis of the average number of cytoplasmic BRCA1 PLA spots per cell is presented in the rightmost columns. ***: p<0.001.
(TIF)

S4 Fig Analysis demonstrating that BRCA1, IFI16, ASC and Caspase-1 are present and interact with each other in the cytoplasm of KSHV *de novo* infected HFF cells. **(A)** Cytoplasmic fractions of primary HFF cells infected with KSHV (30 DNA copies/cell) for 24 h were immunoprecipitated with anti-IFI16, BRCA1 or ASC antibodies and western blotted for IFI16, BRCA1 and Caspase-1. IgG antibodies were used for specificity control in IP reactions. Equal inputs for IPs were assessed by BRCA1, IFI16, ASC and Caspase-1 western blots. Tubulin and TBP western blots were used to confirm purity of the cytoplasmic fractions. **(B and C)** PLA analyses of ASC, IFI16 and BRCA1 associations in KSHV infected HFF cells. Cells were infected with KSHV (30 DNA copies/cell) for 2 h, washed and further incubated for 24 h. Uninfected (B) and infected cells (C) were subjected to PLA reactions with anti-IFI16 and anti-BRCA1 antibodies (middle panels) and anti-IFI16 and anti-ASC antibodies (right panels). After reaction with primary antibodies, cells were washed and reacted with secondary antibodies linked with PLA probes. Secondary antibodies linked with PLA probes without the addition of primary antibodies were used as antibody control (left panels). Red dots indicative of a PLA reaction represent IFI16-BRCA1 complexes (middle panels) and IFI16-ASC complexes (right panels). Yellow arrows indicate cytoplasmic localization of IFI16-BRCA1 and IFI16-ASC complexes in KSHV infected HFF cells.
(TIF)

S1 Table Analysis of protein–protein interaction between IFI16, BRCA1 and DDR proteins. (DOC)
